The article "Ethnomedicinal and folklore inventory of wild plants used by rural communities of valley Samahni, District Bhimber Azad Jammu and Kashmir, Pakistan" was retracted in 2023. Reasons: errors in the data; errors in the methods; errors in the images; duplicated data.

# Ethnomedicinal and folklore inventory of wild plants used by rural communities of valley Samahni, District Bhimber Azad Jammu and Kashmir, Pakistan

**DOI:** 10.1371/journal.pone.0243151

**Published:** 2021-01-13

**Authors:** Muhammad Ishtiaq, Mehwish Maqbool, Muhammad Ajaib, Maqsood Ahmed, Iqbal Hussain, Humaira Khanam, Waheeda Mushtaq, Tanveer Hussain, Shehzad Azam, Khizar Hayat Bhatti, Abdul Ghani

**Affiliations:** 1 Department of Botany, Mirpur University of Science and Technology (MUST), Mirpur, Azad Jammu & Kashmir, Pakistan; 2 Department of Botany, Government College University Faisalabad, Faisalabad, Pakistan; 3 Department of Botany, University of Gujrat, Ahmedabad, Pakistan; 4 Department of Botany, University of Sargodha, Sargodha, Pakistan; University of Poonch Rawalakot, PAKISTAN

## Abstract

The current study describes ethnobotanical (EB) and traditional ethnomedicinal (TEMs) uses of medicinal plants (MPs) of Tehsil Samahni area of Azad Jammu and Kashmir, Pakistan. Indigenous inhabitants of the area mostly reside in remote mountainous areas and depend on wild plants for life necessities and treatment of different diseases. This paper presents first quantitative ethnobotanical study describing the popularity level of MPs in indigenous communities by using relative popularity level (RPL) and rank order of priority (ROP) indices. The data of TEMs and EB uses were collected from 200 interviewees consisting of traditional herbal practioners (110) and farmers (90) from study area using structured and semi-structured interview methodology during year 2019. It was found that illiterate peasants have more knowledge and practice of TEMs than other people. A total of 150 plant species belonging to 58 families with botanical and local names, parts used, mode of recipes preparation, administration mechanism and TEMs uses were documented in systematic manner. It was explored that highest number (7.69%) of plants of Moraceae were used in TEMs and followed by species of Asteraceae (6.29%). The ethnobotanical data was analyzed by using quantitative ethnobotanical tools *viz*: informant consensus factor (ICF), fidelity level (FL), relative frequency of citation (RFC), use value index (UVI), relative importance of plants (RIP), relative populatiry level (RPL) and rank order of popularity (ROP). The leaf ranked first (36.49%) and fruit 2^nd^ (12.07%) being used in TEMs while prevalent use-form was decoction (29.28%), followed by tea (23.05%) and preferably taken as oral (46.66%). ICF analysis proved that diabetes, hypertension, rabies, snake sting and joint pains were the most prevalent occurring infirmities. The highest RFC (0.95) was found for *Acacia modesta*, followed by *Boerhavia procumbens* (RFC:0.87) and *Berberis lycium* (RFC:0.85). The relative importance of MPs was calculated by using UVI and *Moringa oleifera* showed highest (1.38), followed by *Zanthoxylum armatum* (1.25) and *Withania somnifera* (1.24) use-values. High UVI of plants depicts that these species are predominantly used in local health care system. The plants *Phyllanthus emblica*, *Morus macruora*, *Justicia adhatoda* and *Melia azedarach* depicted high values (1.00) of FL and RPL proving that these taxa are commonly used in indigenous medicines by local inhabitants and have better potential for drug discovery by ethnopharmacological analysis. Out of total, 26 species had more than 50% ROP index and *Phyllanthus emblica* and *Flacourtia indica* (ROP = 100) followed by *Morus macruora* (ROP: 97) were used to cure ‘hypertension and hyperlipidemia’ and ‘cough, chest infection’, respectively. It was found that 30% of total species were previously reported as medicinal while 70% plants were first time reported to be used in TEMs and authenticated by using of quantitative ethnobotanical tools. Ethnopharmacological potential of indigenous plants was confirmed by RIP and RPL indices which had been used to cure one or more body systems and were promulgated in the local herbal medicine system. The research provides clues to screen these plant species by using latest phytochemical and pharmacological analysis for novel drug discovery. This study will also be useful for conservation of bioculture traditional knowledge of indigenous communities and the most important is to conserve medicinal plants of the study area for future generations.

The article "Ethnomedicinal and folklore inventory of wild plants used by rural communities of valley Samahni, District Bhimber Azad Jammu and Kashmir, Pakistan" was retracted in 2023. Reasons: errors in the data; errors in the methods; errors in the images; duplicated data.

## Introduction

Plants have been playing a pivotal role in human life because man has been dependent on plants for his requirements and necessities like: food, fodder, fuel, medicines, forage, shelter and aesthetics etc [1–3]. In different regions of world, particularly in rural areas medicinal plants have been utilized to cure and eradicate various diseases and epidemics [4]. About 80% population of the developing countries of world, primarily depends on traditional ethnomedicines (TEMs) or herbal medicines for cure of different diseases [5, 6]. TEMs studies have been of vital significance in discovering of contemporary and targeted allopathic drugs from indigenous medicinal plants (MPs). The ethnobotanical (EB) research on any area provides valuable information about the MPs flora which may be harvested for novel drug discovery through pharmaceutical research [7, 8]. The previous studies provide reference that traditional medical phytonyms’ knowledge has contributed keystone role in development of many vital allopathic drugs from the plants [9, 10].

The article "Ethnomedicinal and folklore inventory of wild plants used by rural communities of valley Samahni, District Bhimber Azad Jammu and Kashmir, Pakistan" was retracted in 2023. Reasons: errors in the data; errors in the methods; errors in the images; duplicated data.

It is estimated that nearly 25% of allopathic medicines have been obtained solely or synergistically from plants and many western drugs are manufactured by using them as ‘model’ production for synthetic and semi-synthetic drugs using dedicated techniques [11]. It is popularized that conventional or allopathic medicines can cause strong side effects if used wrongly whilst herbal or botanic medicines are considered as inexpensive, pure, easily-accessed and safer [12–14].

Pakistan is situated in south Asian region with an area of 884,000 Km^2^ occurring between 25°-38° N, and 62°-76° E. [15]. Azad Jammu and Kashmir territory is one part of whole territory of state of “Kashmir” and it is interesting to narrate that word “Kashmir” means “*land desiccated from water*” whilst Hindu myth states “*Sage Kashyapa drained a lake to produce the land*” [16]. The third group of researchers describe that “*Kashmir is the valley present between the Peer Panjaal mountainous range and great Himalayas*”. The valley is very beautiful, fascinating and Mughal emperor ‘Muhammad Salim Khan’ known as “*Jahanghir”* declared that “*if paradise could be searched in this world anywhere which is Kashmir*”. This predicts that plant biodiversity of Kashmir is un-parallel with any other part of earth [17, 18]. The area of Azad Jammu and Kashmir is 13297Km^2^ with population of 4.2 million. Administratively, Azad Kashmir is divided into ten (10) Districts (administrative units) and Bhimber is one of the districts located at junction with Punjab province. “Etymology of Bhimber” is based on name of its founder/conqueror “Raja Boom Khan” with commemoration as “Bhoom chand” or “Bhoom-pur” and later on, known as “Bhimber” state.

District Bhimber is also called “Bab-e-Kashmir”- the “gateway or door” because it attaches Pakistan with Kashmir and all past time rulers entered in “state of Kashmir” and India (subcontinent) through this city/district. The total area of the district is 1516 Km^2^ which is administratively divided into three subdivisions called Tehsils; Barnala, Bhimber and Samahni [19]. There are different races and people living in it but major ethnic groups are *viz*: Jat, Rajpot, Mirza, Malik, Bhatti, Jaraal, Kashmiri/Bhatt, Awan, Sheikh, Syed and Gojar. The prevalently spoken language is “Hindko” while “Urdu” is known as the *lingua franca* of Bhimber and other parts of AJK; other languages spoken in the area include *viz*: English, Dogri, Kashmiri, Punjabi, Potohari, Saraikee and Pashto [20].

The rationale of study is based on facts that the area under research is mostly mountainous and has many hilly terrains populated by different ethnic groups with specific biocultural paradigm. These indigenous people of the area depend on local plants for their life sustenance and traditional medicines to treat various diseases. The practise of use of herbal or green medicines (GMs) is also well promulgated in different areas of the world. The people of the study area prefer to use TEMs due to cost-effective, accessible, safe and affordable to prepare in home [21, 22]. It is known that approximately 85% traditional medicines used around the globe are botanic in origin prepared from one or more plants species according to folklore recipes [23]. Hence, it is envisaged that MPs are the indigenous phytoheritage or bioheritage and nearly 50, 000 plant species are known for their use in TEMs in different traditional medicine systems of the world [24–26]. Currently, research on traditional herbal medicines is gaining great attention of the world scientific community and in Pakistan many researchers have been working on TEMs of local plants [27–29]. In AJK territory, sporadic research work on TEMs of plant origin have been reported in different ethnobotanical articles [30–33] and on District Bhimber few researchers have conducted the descriptive EB research work [34–40] while hitherto no comprehensive quantitative ethnobotanical research has been conducted on this study area. The present study is focused on documentation of traditional knowledge of indigenous communities of Tehsil Samahni on wild MPs of the area. The purpose of the research was aimed to: (i) to explore and document traditional knowledge of local inhabitants of rural areas about use of wild plants in traditional ethnomedicines (TEMs), (ii) to collect and compile the data of TEMs along with mode of preparation, use-form, parts used, folklore recipes used by local herbalists, (iii) to authenticate the data of TEMs by using quantitative tools like RPL, ROP, ICF, UVI, FL and RFC in order to explore the most prevalently used species in TEMs and to recommend it for further ethnopharmacological screening for drug discovery and development and (iv) to give recommendations for conservation of wild medicinal plants endemic in the area.

The article "Ethnomedicinal and folklore inventory of wild plants used by rural communities of valley Samahni, District Bhimber Azad Jammu and Kashmir, Pakistan" was retracted in 2023. Reasons: errors in the data; errors in the methods; errors in the images; duplicated data.

## Materials and methodologies

(flowchart of methodology is presented in Fig 2).

### Description of the study area

Azad Jammu Kashmir state is divided into ten administrative units called Districts and Bhimber is one of these districts. Edaphologically it is linked with Gujrat (Pakistan) on south, Mirpur western-side while on eastern and north-east side it is linked with Indian Kashmir (District Jammu and Rajori) and on north-west is District Kotli. It demarcates that area has diverse bioculture and different communities reside in the area. So, due to unique geographic location of District Bhimber; the area is archaeologically very rich with cultural amalgam of different regions and ethnicity of the past eras (Fig 1). To visit the Kashmir valley, the Mughal Emperors usually used this route passing through the area for travelling [41]. The current research project is conducted in subdivision Samahni of District Bhimber of AJK. Geographic coordinates describe that Bhimber is located between latitude 32–48 to 33–34 and longitude 73–55 to 74–45 degree with area of 1516 Km^2^, altitude of 1118 ft from sea level inhabitating population of ca. 4500,000 [42].

**Fig 1:** Map of study area Tehsil Samahni (District Bhimber) of Azad Jammu & Kashmir, Pakistan.

Bhimber city has distance of 50 Km from Mirpur, 48 Km from Gujrat (Pakistan) 166 Km Islamabad (Pakistan) and 241 Km from Srinagar (Indian Occupied Kashmir) [43]. Bhimber is located in hub or lap of Shiwalik mountainous range with high rainfall in Feb-March but peak is seen in monsoon season (July to August). The average rainfall is ca.1233 mm per month and hailing occurs in months of February and July [44]. Temperature of the area ranges upto 45°C in summer (May-June) while remains cold in winter and humidity content usually is high during rainy and winter seasons (69%) [44]. Anthropological survey describes that the area has diverse ethnicity and famous casts residing include *viz*: Jat, Mirza, Malik, Rajpot, Bhati, Sheikh, Syed and Gojars while Jat and Rajpot are main ethnic groups having high population and land resources [45]. Other minorities use land of these big tribes for agriculture purpose because they have very little land of their own. Many people live in mountains and/or near mountains, so they get their needs of food, fodder, construction wood and fuel from natural resources (forests) [46]. According to one point of view historians “*Kashmiri people*” belong to one ancestral ethnic group called “*Dardic”* who was known as Indo-Ayran prevalently living in east-border of Afghanistan and northern areas of Pakistan and India. Currently, 90% population of Bhimber has “Punjabi” ancestors with closest religious, cultural and geographical relations to Potohar-belt inhabitants [47, 48]. The commonly spoken language is “*Hindko or Saraeki*” which is influenced by Punjabi language due to its neighborhood and the known languages spoken consist of: Urdu, English, Dogri, Kashmiri, Punjabi, Potohari, Saraikee and Pashto. Pashto is also used by migrant Afghan communities who came here in 1989–90, known as “*War Displayed Persons (WDPs*)” as shown in map of study area (Fig 1) and now living here in District Bhimber to earn their livelihood [45].

The article "Ethnomedicinal and folklore inventory of wild plants used by rural communities of valley Samahni, District Bhimber Azad Jammu and Kashmir, Pakistan" was retracted in 2023. Reasons: errors in the data; errors in the methods; errors in the images; duplicated data.

### Ethnomedicinal data compilation and authentication

Ethnomedicinal use data of wild medicinal plants was gathered from the local informants using structured and semi-structured interview methodology with documentation of the information in questionnaire form during year-2019 (Fig 2). About 200 informants comprising of both male (120) and female (80) were involved in the study and during all trips one male and one female guide or translator was accompanied because rural and mountainous people use different languages and dialects, hence it was very important to use indigenous translator to know the real knowledge about indigenous flora from the native communities [49–52]. The interviewees were farmers, house-women, midwives, herbalist and traditional phytotherapist (TPT) while it has been seen that most of the people were illiterate or had very basic education and only few had graduation level literacy; thus extracting diverse and maximum knowledge of TEMs from the indigenous communities. In the research trips not only traditional knowledge of TEMs was documented but also plant specimens were collected with guidance of local people describing their native names and tonic preparation methods were narrated in field notebook. For this study, interviewees were selected gender free manner and each collected plant was showed to “five or more” individuals and asked to tell their ethnomedicinal, ethnobotanical uses and occurrence place with population density of each species. In this procedure, if same data or information about the species was described by three or more than three persons (>60%) then it was declared “authentic” and included in the study for better reliability and further research analysis. However, the less information collected about certain plants does not mean that they are of less significance in TEMs, that might be due to reason that traditional ethnomedicinal knowledge (TEK) about wild plants is gradually disappearing in younger generations or population of the plants is becoming scarce day by day due to various threatening factors [53, 54]. For proper authentication of the ethnomedicinal data, the botanical and local names with family of each plant were verified manually with herbarium specimens, taxonomic literature (hard and soft form), manuals, Flora of Pakistan and cross checked with online data from the plant list website or flora of Pakistan & litrature [55–59]. All collected plants were brought under standardized voucher numbering system with labels and cross-referenced with field notebook (FNB) record to further validate their authenticity [60–62]. All gathered ethnomedicinal data of plants was presented in alphabetical order comprising of botanical names, common names, family, plant parts, preparation mode, administration method, diseases cured and other ethnobotanical uses promulgated in the study area. During the field surveys, plants specimens were collected properly (having flowers, fruit or both) and preserved according to the standard process for herbarium (MUH) [47, 63]. The herbarium specimens were prepared according to protocol of previous researchers like Seshagirirao *et al*., (2016), Vitalini *et al*., (2013) and Ishtiaq *et al*., (2010a) [39, 64, 65] and deposited in the herbarium of the Department of Botany with proper voucher number allotment for future reference because they will assist taxonomy students and researchers to identify the required species for further collection from same and/or other areas of the study area and Azad Kashmir regions [66, 67]. The collected plant specimens were properly identified using Flora of Pakistan data “www.eflora.com”, the plant list “www.theplantlist.org” and comparing with printed Flora book [68, 69]. Whereas another website named “International Plant Name Index” with webpage “www.ipni.org” was used for cross checking of botanical and family names of the plants [70]. The collected plants were identified by Dr. Muhammad Ajaib; a taxonomist of the Department of Botany and all prepared herbarium vouchers bearing code “MUH-”, were kept in herbarium, Department of Botany Mirpur University of Science and Technology (MUST), Bhimber Campus, AJK, Pakistan for future reference.

The article "Ethnomedicinal and folklore inventory of wild plants used by rural communities of valley Samahni, District Bhimber Azad Jammu and Kashmir, Pakistan" was retracted in 2023. Reasons: errors in the data; errors in the methods; errors in the images; duplicated data.

**Fig 2:** 

### Ethical statement

The official permission of plan regarding field study and collection of plants from wild areas and Forest zones of Samahni, District Bhimber of AJK was obtained from departmental ethical committee (DEC) duly counter signed by convener of institutional ethical committee.

### Field permit number of field study

The study of plants and their collection from wild forest areas of Samahni (AJK) for experimental and herbarium specimen preparation was prior approved from the concerned head of Forest Department with proper permit number vide: DFO/1277/2019; dated: 02/01/2019. The right of obedience of forest rules was fully followed as per SOPs provided by the relevant office.

### Quantitative analysis

In the research, quantitative ethnobotanical (EB) and ethnomedicinal (EM) data was collected through questionnaire process, tabulated in matrix form and analysed through statistical tools following methodology of previous ethnobotanists (Cook, 1995; Amjad *et al*., 2017; Ishtiaq *et al*., 2013b) [47, 54, 57, 71]. Stringent scrutiny was applied for extraction and compilation of the authentic information about the flora of District Bhimber of AJK. The authenticity, replicability and reliability of collected EB and EM information were rechecked by using the following microstatistical tools like: “informant consensus factor” (ICF), “fidelity level” (FL), “relative importance of plant” (RIP), “use value index” (UVI), “relatvie frequency of citation” (RFC), “relative popularity level” (RPL) and “rank order of priority” (ROP) following the procedures previous researchers like Ishtiaq *et al*., (2007b) and Mesfin, *et al*., (2009) [61, 71, 72].

The article "Ethnomedicinal and folklore inventory of wild plants used by rural communities of valley Samahni, District Bhimber Azad Jammu and Kashmir, Pakistan" was retracted in 2023. Reasons: errors in the data; errors in the methods; errors in the images; duplicated data.

### Informant consensus factor (ICF)

Informant consensus factor was calculated for every category or group of diseases to determine the consensus value of informants on the reported ethnomedicinal uses for the group of diseases and later on various infirmities were categorized in different groups. ICF was calculated by the following formula:

$$\text{ICF}=\frac{\text{N}ur-{\text{N}}_{t}}{\text{N}ur-1}$$

where N_ur_ is number of use citations in each category/group minus (-) N_t_ that is total number of plant species used; divided (/) by the number of use citations in each category minus one as per given formula above [57, 73–75]. This maximum value in ICF is one (01), if experimental values are one or near to one then it means that reported plant species are prevalently used by major part of the local communities confirming their authenticity regarding the ailments’ cure. If ICF value is zero (0) or near to zero then it confirms that local people randomly use the plant (s) to treat the cited infirmity [57, 62, 76].

### Fidelity level (FL)

The fidelity level of the data was calculated which depicts the percentage (%age) of interviewees claiming any use of a particular plant for the same major purpose or field and total number of commonly reported usages or ailments. It was calculated according to formula:

$$\text{FL}(\%)=\frac{\text{Np}}{\text{N}}\times 100$$

whereas; N_p_ depicts number of informants, who claimed a particular use of a plant species used for a typical disease and N means that number of informants/interviewees who used the plants as an ethnomedicine to treat given diseases [57, 77, 78].

### Relative popularity level (RPL)

The relative popularity level index of the plants was calculated to assure and re-affirm obtained FL statistical values of the plants. Sometime, FL cannot be explained properply, particulalry when it provides similar values although above 50%, then there is need of a correction factor and RPL is used for this purpose. RPL usually ranges between 0–1 showing lowest and highest range. If its value is one or near to it, then it proves that plant species is frequently used to cure the disease and vice versa [62, 79–81]. It is known that number of uses increases when number of informants rises because of correlation coefficient factor r = 0.10. For example, if one plant species is cited by more 25 or more informants as ethnomedicines then its RPL rank is raised and RPL is determined as percentage of (I_u_ /25); score one (1) is assigned if cited or mentioned by the half or more number (12) of total informants that was 25 and plant species used to cure any disease is known as popular (“P”) medicinal plant in the area. If any plant is cited by less than 12 informants then RPL value will be ranked as unpopular (“UP”) [62, 82]. The marginalized value between ‘P and UP’ of the plant is the point where if informants number is increased then number of medicinal uses per plant species does not rise.

The article "Ethnomedicinal and folklore inventory of wild plants used by rural communities of valley Samahni, District Bhimber Azad Jammu and Kashmir, Pakistan" was retracted in 2023. Reasons: errors in the data; errors in the methods; errors in the images; duplicated data.

### Rank order popularity (ROP)

ROP is used as correction factor when FL and RPL vlaues were different from each other and for proper rank order determination. The ROP was calculated by using formula *ROP* = *FLxRPL*, where ROP value depicts high level or order of popularity of MPs in the specific disease [62, 83]. These two tools (RPL and ROP) of EB study are commonly used for determination of usefulness of different MPs to cure diseases in the local area by indigenous communities.

### Use value index

The use value index (UVI) demarcates relative importance of different uses of the specific species. It was determined by using past cited formula following Vijayakumar *et al*., (2015) protocol [62, 84].

$${\text{UV}}_{\text{i}}=\frac{\Sigma {\text{U}}_{\text{i}}}{\text{N}}$$

whereas UV indicates “relative use value” of the single species; “U” is the ‘number of uses mentioned by each informant for the species and “N” is the ‘total number of informants who reported that species.

### Relative frequency of citation (RFC)

Relative frequency of citation is used an index to explore significance or importance of each species occurring in the local area. RFC was determined by “dividing the number of informants” confirming the frequency of citation (FC) by “total number of informants” who participated in survey according formula of Vijayakumar *et al*., (2015) [62, 84–86].

$$\text{RFC}=\frac{\text{FC}}{\text{N}}$$

whereas ‘0 < RFC >1’; and FC is the ‘number of informants’ reporting use of a particular species and N is the ‘total number of informants’ involved in study survey.

### Relative importance of plant (RIP)

The pharmacological or pharmaceutical significance of each plant in local culture was determined by using relative importance (RIP) term and it was determined by the following formula as following protocol of Umair *et al*. [62] and Amjad *et al*. [59].

$$\text{RIP}=\frac{\text{Rel}.\;\text{Ph}+\text{Rel}.\;\text{B}.\text{S}.\times \text{100}}{\text{2}}$$

whereas Ph. is pharmacological features of the plants and Rel. Ph. is relative pharmacological importance; rel. BS is body system treated. The relative Pharmacological significance can be caluclated by the given below formula.

$$\text{rel}.\text{Ph}=\frac{\text{Ph}.\;\text{of}\;\text{given}\;\text{Plant}}{\text{Ph}\;\text{of}\;\text{all}\;\text{reported}\;\text{plant}\;\text{species}}$$

whereas Ph. is pharmacological attributes of the each provided plant and rel. Ph. is the relative number of pharmacological properties referenced for an individual plant.

$$\text{rel}.\text{BS}=\frac{\text{BS}\;\text{of}\;\text{given}\;\text{Plant}}{\text{BS}\;\text{of}\;\text{all}\;\text{reported}\;\text{plant}\;\text{species}}$$

whereas BS is the number of body system healed by single species and rel. BS is relative number of body system treated by the given plant species.

The article "Ethnomedicinal and folklore inventory of wild plants used by rural communities of valley Samahni, District Bhimber Azad Jammu and Kashmir, Pakistan" was retracted in 2023. Reasons: errors in the data; errors in the methods; errors in the images; duplicated data.

## Results and discussion

### Demographic features of the informants

In this study ethnomedicinal and ethnobotanical information of 150 local plants from Samahni valley of District Bhimber of AJK was collected from 200 local informants who consisted of two types (i) 110 traditional herbal therapists (THP) and 90 indigenous people (IP) from different villages and local markets. The demographic information was fractionated into different categories which are presented Fig 3. In the survey, it was found that mostly male informants have more knowledge of TEMs than female respondents. The reason of this difference may be due the fact that male can easily learn education of TEMs from ancestors and also male are more friendly in dissemination of traditional ethnomedicinal knowledge (TEK) about the local plants than female practitioners. Secondly, females of the rural areas were reluctant and shy in information sharing due to conventional family cultural and religious customs of the area [87]. It was found that traditional herbal practioners (THPs) have more information of TEK about the wild MPs than laymen or farmers. The indigenous people (IP) who comprises of various subgroups such as farmers, midwives, teachers, house-wives and shepherds also depicted good amount of TEK but have restricted approach for proper identification of wild MPs of the area as per scientific criterion; however they knew all or maximum local names of the plants. They use MPs not only at their own homes as food phytonyms and tonics but also sale to herbal doctors and local markets traders to earn money. It was seen that THPs with experience of 10–15 years had highest (33%) TEMs knowledge, followed by experience group of 15–20 years (16.6%). It was found that illiterate people had more information of TEMs because they follow traditional cultural rituals more prevalently with great passion and belief than educated inhabitants [46, 87]. A common trend was seen that with rise of education level, there was decline in TEK and use of TEMs that may be due to fact that literate people prefer to use allopathic medicines because they can afford to buy these medicines and prefer prompt relief from infirmities. It was also found that old people have more information about the MPs and TEMs than young community because they spent long time with their ancestors and used TEMs for disease cure [46]. It was seen that indigenous old and illiterate communities have more belief or trust in TEMs and use of MPs in their daily to cure different infirmities and similar studies had been cited in the past studies in Azad Kashmir [1, 3, 6, 15, 59, 117], Pakistan [2, 4, 83, 114] and other countries as well [21, 88, 89].

The article "Ethnomedicinal and folklore inventory of wild plants used by rural communities of valley Samahni, District Bhimber Azad Jammu and Kashmir, Pakistan" was retracted in 2023. Reasons: errors in the data; errors in the methods; errors in the images; duplicated data.

**Fig 3:** Informants data depicting the demographic features in Valley of Samahni, AJK, Pakistan.

### Family index depicting distribution patterns of medicinal plants

The study revealed ethnomedicinal and ethnobotanical uses of 150 plants being promulgated by indigenous people of the area. These plants belonged to 58 families with Moraceae had highest value (7.69%), followed by Asteraceae with 6.29%, Poaceae and Euphorbiaceae 5.59% each (Table 1).

**Table 1:** Family index depicting distribution of medicinal plants in Samahni Area of AJK.

Name of Family	No of Species	%age contribution	Name of Family	No of Species	%age contribution
Acanthaceae	01	0.70	Lamiaceae	07	4.90
Anacardiaceae	01	0.70	Loranthaceae	02	1.40
Asclepiadaceae	02	1.40	Malvaceae	05	3.50
Amaranthaceae	05	3.50	Meliaceae	03	2.10
Alliaceae	01	0.70	Mimosaceae	03	2.10
Apocynaceae	03	2.10	Moraceae	11	7.69
Asphodelaceae	01	0.70	Moringaceae	01	0.70
Asteraceae	09	6.29	Myrtaceae	01	0.70
Arecaceae	01	0.70	Nyctaginaceae	01	0.70
Berberidaceae	01	0.70	Oleaceae	01	0.70
Bombacaeae	01	0.70	Oxalidaceae	01	0.70
Boraginaceae	03	2.10	Pinaceae	01	0.70
Brassicaceae	02	1.40	Plantaginaceae	01	0.70
Caesalpiniaceae	02	1.40	Papaveraceae	02	1.40
Caryophyllaceae	02	1.40	Papilionaceae	07	4.90
Capparaceae	02	1.40	Phyllanthaceae	01	0.70
Chenopodiaceae	01	0.70	Poaceae	08	5.59
Celastraceae	01	0.70	Polygonaceae	02	1.40
Colchicaceae	01	0.70	Portulacaceae	01	0.70
Combretaceae	01	0.70	Ranunculaceae	04	2.80
Commelinaceae	01	0.70	Rosaceae	01	0.70
Convolvulaceae	05	3.50	Rutaceae	01	0.70
Cuscutaceae	01	0.70	Salicaceae	02	1.40
Cucurbitaceae	01	0.70	Scrophulariaceae	02	1.40
Cyperaceae	02	1.40	Solanaceae	07	4.90
Euphorbiaceae	08	5.59	Tiliaceae	02	1.40
Flacourtiaceae	01	0.70	Urticaceae	01	0.70
Fumariaceae	01	0.70	Violaceae	01	0.70
Juglandaceae	01	0.70	Zygophyllaceae	01	0.70

These above stated families are the most prevalent and dominant in the study area proving that MPs of these families are prevalent in the area and easily accessible to the local communities. The prevalence of these families in TEK of the area means that plants of these families have good quantity of phytoconstituents and local inhabitants have been using these for long time. The remaining families having ≤ five or less number of plants are also being used in TEMs but their ratio is less indicating either their less popularity or scare occurrence in the area. Similar reports about the presence of secondary metabolites have been cited in the previous works where plants of families like Moraceae, Lamiaceae, Asteraceae and Poaceae have been used for cure of different infirmities by local people of KPK, areas of Pakistan [90]. Many plant species reported from the study area have been used for cure of diabetics, respiratory disorders, skin allergies, stomachache and other infirmities (Tables 2 and 3). In previous research studies, similar results have been reported that many plants belonging to 46 families of lesser Himalaya regions of Pakistan are prevalently used to cure reproductive and respiratory disorders [91]. Another researcher, Kayani (2014) had conducted research work on TEMs uses of 120 plans belonging to fifty one families which had been used by indigenous people of the Abbottabad, KPK of Pakistan [92]. The plants cited here from the study area have been used by local rural communities as TEMs and these findings are in congruent with previous ethnobotanical works of many researchers [93–97]. The plants which have perennial life pattern showed more use in TEMS than annual species because their leaves, roots and fruits are prevalently available for use as ethnomedicines [98–100].

The article "Ethnomedicinal and folklore inventory of wild plants used by rural communities of valley Samahni, District Bhimber Azad Jammu and Kashmir, Pakistan" was retracted in 2023. Reasons: errors in the data; errors in the methods; errors in the images; duplicated data.

**Table 2:** Informant consensus factor (ICF) by categories of diseases in study area of Samahni, Azad Jammu and Kashmir, Pakistan.

S No	Category/ Plants Used for Disease(s)	Species	(%) All species	Use citations	(%) All citations	ICF (nur-nt)/ (nur-1)
1	Diabetics and blood pressure	20	08.29	330	15.50	0.94
2	Fever, flu, headache, bronchitis, cough	45	18.67	255	11.97	0.82
3	Epilepsy and mental disorders	34	14.10	211	09.91	0.84
4	Stomachic, constipation, haemorrhoids	28	11.61	196	09.20	0.86
5	Jaundice, spleen and liver disorders.	42	17.42	245	11.50	0.83
6	Cardiovascular disorders	18	07.46	158	07.42	0.89
7	Rabies and other sting pains	14	05.80	190	08.92	0.93
8	Gut, tuberculosis, ulcers and leucorrhea	19	07.88	181	08.50	0.90
9	Arthritis and joint disorders	22	09.12	235	11.03	0.91
10	Kidney and urinary disorders	19	07.88	128	06.01	0.85

**Table 3:** Relative frequency of citation (RFC) and use value index (UVI) of the most commonly used indigenous plants by the local people of different areas of Samahni, District Bhimber (AJK), Pakistan.

S. No	Botanical Names with Family	Local Name	Flowering Period	Life Habit/ Life Form			Part(s)/Form (s) of Usage	Application mode	Phytotherapeutic Utilization as EMs and Phytonyms	RFC	UV	ƩUI	UVI
										(with 55 Informants in the Analysis)			
1.	*Acacia modesta* Wall. Leguminosae; subfamily Mimosaceae MUH-1366	Phulaai	Mar. to May	W	T	P	Bark, Gum, leaf/decoction, tea	Oral, gargle and topical	Toothache, cough dysentery, bacterial infections, stimulant, backache, venereal infirmities and leprosy.	52	0.95	48	0.87
2.	*Acacia nilotica* (L.) Delile M. Leguminosae; subfamily Mimosaceae MUH-1368	Kikar	Mar. to Aug.	W	T	P	Bark, Gum/Decoction, powder	Oral, gargle and topical	Wound healing, fever, cough, cold, toothache, feet infection, sexual disorders, diabetics, body weakness and used as ethnoveterinary medicines (EVMs).	22	0.40	43	0.78
3.	*Achyranthus aspera* L. Amaranthaceae MUH-1539	Phutkanda	Feb. to Apr.	W	H	A	Fruit, leaf, seed /Decoction, powder	Oral and topical	Urinary diseases, asthma, stomachache, fever, cough, constipation, diuretic, wound healing, bacterial infections and prolapse problems of cattle as EVMs.	22	0.40	38	0.69
4.	*Aerva sanguinolenta* (L.) Blume Amaranthaceae MUH-1544	Chti boti	Mar. to Sep.	W	H	A	Leaf, root, stem, flower/ extract, tea	Oral, and topical	Diabetics, skin infection, bacterial and fungal disease wound, bleeding bruises healer, chest infections, edema, inflammation, snake bite, dermatitis and allergy.	12	0.22	41	0.75
5.	*Ajuga bracteosa* Wall ex Benth. Lamiaceae MUH-1529	Haree booti	Mar. to Dec.	W	H	A	Leaf, bark / Powder, juice	Oral, and topical	Hypertension, jaundice, sore throat and ulcer.	34	0.62	44	0.80
6.	*Albizia lebbeck* (L.) Benth. Leguminosae; subfamily Mimosaceae MUH-1370	Cheeta Shreen	May to Jun.	W	T	P	Bark, Seed/ Powder, decoction	Oral, and topical	Kidney disorders, wormicide and skin allergy.	28	0.51	33	0.60
7.	*Allium jacquemontii* Kunth Alliaceae MUH-1608	Jangli Piaz	Mar. to May	W	H	A	Leaf, bulb/Juice, extract	Oral, and topical	Snake bite, sting of scorpion and other poisonous insects and used as EVMs.	24	0.44	46	0.84
8.	*Aloe vera* (L.) Burm. f. Asphodelaceae MUH-1612	Kawal Gandal	Jan. to Apr.	W	H	A	Leaf, bulb/Juice, tea, decoction	Oral and topical	Piles, anal irritation, diabetics, baldness, wound healing, skin diseases, cancer, cardiovascular diseases and used as EVMs.	34	0.62	52	0.95
9.	*Alternanthera pungens* L. Amaranthaceae MUH-1541	Taahee booti	Apr. to Nov.	W	H	A	Whole plant/powder, juice	Oral and topical	Diuretic issues, cancer, eye related diseases, anemia and wound healing.	24	0.44	46	0.84
10.	*Amaranthus viridis* L. Amaranthaceae MUH-1537	Chulair	All the year	W	H	A	Leaf, root/Juice, decoction	Oral, and topical	Stomachache, constipation and edema.	23	0.42	47	0.85
11.	*Artemisia scoparia* Waldst. & Kit. Asteraceae MUH-1429	Kaalee booti	Jun. to Dec.	W	H	A	Leaf, root/Juice, infusion	Oral, and topical	Constipation, depurative and toothache.	35	0.64	43	0.78
12.	*Artemisia vulgaris* L. Asteraceae MUH-1430	Kaali buti	Jun. to Dec.	W	H	A	Leaf, bark/Juice, tea	Oral and topical	Malarial diseases, asthma, diarrhea, nervous, febrifuge and tonic.	32	0.58	43	0.78
13.	*Azadirachta indica* A. Juss. Meliaceae MUH-1321	Neem	Mar. to May	W	T	P	Seed, leaf, bark/ juice, decoction	Oral and topical	Diabetics, intestinal worms, blood purification, microbial diseases, wounds and used as EVMs.	37	0.67	57	1.04
14.	*Bauhinia variegata* L. Leguminosae; subfamily Caesalpiniaceae MUH-1363	Kalyar	Feb. to Apr.	W	T	P	Flower, buds, leaf/Powder, tea, infusion	Oral and topical	Stomach diseases, bacterial infections, dysentery, hemorrhoids, piles, laxative, wound healing, tumor and snake poison.	31	0.56	43	0.78
15.	*Berberis lycium* Royle. Berberidaceae MUH-1289	Sumbalo	Apr. to Jun.	W	S	P	Leaf, bark/Juice, tea	Oral and topical	Dysentery, hypertension, liver disorders, wound healing, Jaundice, dyspepsia, sore throat and itching.	52	0.95	52	0.95
16.	*Boerhavia procumbens* Banks ex Roxb. Nyctaginaceae MUH-1535	Sanaati	All the year	W	H	A	Leaf, root, whole plant/ tea, decoction	Oral and topical	Dysentery, stomachache and aphrodisiac.	48	0.87	54	0.98
17.	*Bombax ceiba* L. Bombacaeae MUH-1302	Simbal	Feb. to Apr.	W	T	P	Leaves, flower/ infusion, powder	Oral and topical	Cough, fever, menstrual pain, flu, sore throat and tumors.	36	0.65	40	0.73
18.	*Bromus japonicus* L. Poaceae MUH-1658	Lomar gasss	Jul. to Aug.	W	H	A	Leaf, whole plant/Extract	Oral and topical	Chest pains and edema or inflammation issues.	21	0.38	22	0.40
19.	*Butea monosperma* (Lam.) Taub. Leguminosae; subfamily Papilionaceae MUH-1337	Cheechra	Mar. to May	W	T	P	Stem, Fruit/ powder, tea, infusion	Oral and topical	Eye diseases, diabetes and kidney disorders.	23	0.42	40	0.73
20.	*Calotropis procera* (Aiton) Dryand. Asclepiadaceae MUH-1448	Aak	All the year	W	S	P	Flower, latex, leaf/Paste, extract	Oral and topical	Asthma, cough, fever, wound healing, snake bite, skin diseases, fungus diseases, scabies and used as EVMs.	41	0.75	41	0.75
21.	*Capparis decidua* (Forssk.) Edgew. Capparaceae MUH-1583	Kareer	Mar. to Apr.	W	S	P	Leaf, stem, root, bark/Decoction, tea	Oraland topical	Bacterial diseases, cough and flu.	34	0.62	46	0.84
22.	*Capparis sepiaria* L. Capparaceae MUH-1584	Kareere	Mar. to Apr.	W	S	P	Leaf, stem, root, bark/ Decoction, tea	Oral and topical	Bacteria and fungi infections, foot or skin allergy.	35	0.64	42	0.76
23.	*Carissa opaca* Stapf ex Haines. Apocynaceae MUH-1444	Ganranda	Apr. to Jun.	W	S	P	Latex, fruit, leaf/ Juice, infusion, tea	Oral and topical	Snake and scorpion bite, stomachache, jaundice and hepatitis.	44	0.80	51	0.93
24.	*Cuscuta reflexa* Roxb. Cuscutaceae MUH-1482	Kaash bail	Aug. to Sep.	W	H	A	Stem/ juice, infusion	Oral and topical	Lice killer, skin diseases, anemia and weakness in children.	33	0.60	45	0.82
25.	*Casearia tomentosa* Roxb. Salicaceae MUH-1290	Chillah	Mar. to Jun.	W	T	P	Fruit, leaf/ extract, infusion	Oral, and topical	Fish killer/ catching used as bio-net, diabetic and urinary disorders.	16	0.29	32	0.58
26.	*Cassia fistula* L. Leguminosae; subfamily Caesalpiniaceae MUH-1364	Krinjal	Apr. to May	W	T	P	Leaf, seeds, pods/ tea, powder, infusion	Oral and topical	Stomach problem, asthma, febrifuge and as source ethnoveterinary medicines (EVMs).	32	0.58	34	0.62
27.	*Cenchrus biflorus* Roxb. Poaceae MUH-1637	Bhurat Gass	Jan. to Apr.	W	H	A	Leaf, whole plant/ extract, tea	Oral and topical	Seeds edible, bacterial diseases, chest infection and cough.	32	0.58	35	0.64
28.	*Ceropegia bulbosa* L. Asclepiadaceae MUH-1453	Galot	Jul. to Sep.	W	H	A	Leaf, tuber/Paste, juice, tea	Oral and topical	Spleen and kidney disorders, cancer, gasteroprotective, microbial infections and inflammatory issues.	34	0.62	42	0.76
29.	*Chenopodium album* L. Chenopodiaceae MUH-1545	Bathoo	Jan. to Sep.	W	H	A	Leaf, root/Juice, paste, infusion	Oral and topical	Constipation, laxative and stomach pains.	32	0.58	46	0.84
30.	*Chenopodium ambrosiodies* L. MUH-1546	Gandee buti	May to Oct.	W	H	A	Leaf, root/ Juice, paste, infusion	Oral, and topical	Wound healing, stomach wormicidal, constipation and piles.	27	0.49	42	0.76
31.	*Cichorium intybus* L. Asteraceae MUH-1402	Kasni	Jun. to Sep.	W	H	A	Leaf, seeds/ powder, extract	Oral, gargle and topical	Fever, indigestion, omititng. blood purifier, kideny problems, urinary problems, hapatitis and tooth pains.	32	0.58	32	0.58
32.	*Cirsium arvensis* (L.) Scop. Asteraceae MUH-1435	Kandyaree	Mar. to May	W	H	A	Leaf, root, flower/extract, powder	Oral and topical	Bacterial and fungal diseases or infections, cough and flu.	30	0.55	42	0.76
33.	*Citrullus colocynthis* (L.) Shard Cucurbitaceae MUH-1388	Tuma	Jan. to Apr.	W	H	A	Lea, fruit, seed/ powder, decoction	Oral and topical	Emmenagogue, purgative, cathartic, amenorrhea, syphilis, tumors, diabetics, jaundice, rheumatism, urinary problems and snake bite. The plant is also used as ethnoveterinary medicines (EVMs).	36	0.65	41	0.75
34.	*Clematis grata* Wall. Ranunculaceae MUH-1261	Bohree bail	Apr. to Aug.	W	L	A	Leaf, stem, bark/ paste, infusion	Oral and topical	Body weakness & slimness in childeen and wormicide in goats and animals.	25	0.45	18	0.33
35.	*Clematis graveolens* Lindl. Ranunculaceae MUH-1262	Baileree	Apr. to May	W	L	A	Leaf, root/ extract, decoction	Oral and topical	Wormicidal in animals, and to cure tumors or boils.	25	0.45	45	0.82
36.	*Clematis connata* DC. Ranunculaceae MUH-1263	Clemoo, bailary	Jul. to Aug.	W	L	A	Leaf and bark/ tea, decoction	Oral and topical	To elelminate stomach worms in animals, cure boils and tumors.	21	0.38	35	0.64
37.	*Colebrookea oppositifolia* Smith. Lamiaceae MUH-1519	Bindaa	Jan. to Apr.	W	H	A	Leaf, bark, root/ powder, extract	Oral and topical	Fever, flu, wounds, bruises cure and epilepsy.	36	0.65	35	0.64
38.	*Commelina benghalensis* L. Commelinaceae MUH-1617	Surkara	Aug. to Nov.	W	H	A	Leaf, whole plant/Juice, extract	Oral and topical	Constipation, diuretic, febrifuge, treat burns and inflammatory issues.	24	0.44	42	0.76
39.	*Convolvulus arvensis* L. Convolvulaceae MUH-1470	Harn kuree	Feb. to Aug.	W	H	A	Leaf, whole plant/Extract, juice	Oral and topical	Diuretic and purgative, fever, loss of memory and fatigue.	14	0.25	24	0.44
40.	*Convolvulus prostratus* Forssk. Convolvulaceae MUH-1471	Lailee	Feb. to Aug.	W	H	A	Leaf, whole plant/Juice, infusion	Oral and topical	Fever, nervous debility, and loss of memory, purgative and body fatigue/muscle pains.	16	0.29	32	0.58
41.	*Corchorus olitorius* L. Tiliaceae MUH-1309	Jangli Patsan	May to Jul.	W	H	A	Leaf, WP/ powder, juice	Oral and topical	Ascites, dysuria pain, cystitis, fever piles and tumors.	22	0.40	28	0.51
42.	*Cordia gharaf* (Forssk.) Ehren. ex Asch Boraginaceae MUH-1462	Gondee	Apr. to Jun.	W	T	P	Leaf, root, Stem/ juice, tea, powder	Oral and topical	Fever, cough, chest infection, diuretic, demulcent and stomachache.	32	0.58	44	0.80
43.	*Cordia obliqa* L. Boraginaceae MUH-1461	Lasoora	Mar. to Apr.	W	T	P	Whole plant/ pickle, juice, tea	Oral and topical	Diuretic, fever, joints pain, dry cough, throats pain, tonic and stomach ulcer.	35	0.64	51	0.93
44.	*Cymbopogan citratus* (John) Schutt Poaceae MUH-1468	Lemon gass	Oct-Dec.	W	H	A	Leaf, whole plant/ tea	Oral and topical	Flu, amoebic diseases, bacterial infection, diarrhea, fungal infirmities, inflammations and cough.	13	0.24	32	0.58
45.	*Cynodon dactylon* (L.) Pers. Poaceae MUH-1645	Khabal gass	All the year	W	H	A	Whole plant / extract, tea	Oral and topical	Wound healing, skin diseases, fever and respiratory disorders.	22	0.40	54	0.98
46.	*Cynoglossum lanceolatum* Forssk. Boraginaceae MUH-1469	Lahndara	Jun. to Sep.	W	H	A	Leaf, bark / extract, tea, infusion	Oral and topical	Flu, cough, heart issues, asthma and fever.	32	0.58	44	0.80
47.	*Datura innoxia* Mill. Solanaceae MUH-1489	Datoora	May to Oct.	W	S	P	Fruit, leaf/ powder, decoction	Oral and topical	Insecticidal, baldness, wound healing, antiseptic, sedative, narcotic, asthma and mosquito repellant.	34	0.62	51	0.93
48.	*Datura stramonium* L. Solanaceae MUH-1490	Tatoora	May to Jul.	W	S	P	Leaf, fruit, root/powder, decoction	Oral and topical	Insecticide, antipyretic, narcotic, verimicidal, cold and fever in cattle as EVM. It is used for early copulation and pregnancy in cow/ buffaloes.	36	0.65	50	0.91
49.	*Digera muricata* (L.) Mart. Amaranthaceae MUH-1536	Toondola	July-Dec	W	H	A	Leaf, whole plant/ tea, infusion	Oral and topical	Digestive disorders and urinary problems.	22	0.40	23	0.42
50.	*Echinochloa colona* (L.) Link Poaceae MUH-1656	Mordhaani	Mar to Jul.	W	H	A	Leaf, root/ juice, paste	Oral and topical	Dropsy treatment, skin rashes, spleen enlargement, hemorrhage and irritations.	15	0.27	17	0.31
51.	*Echinochola crus-galli* L. Poaceae MUH-1658	Cockspur grass	Mar to Jul.	W	H	A	Leaf, whole plant/paste, extract	Oral and topical	Spleen disorders, fever, skin allergies and cough.	34	0.62	45	0.82
52.	*Echinops echinatus* Roxb. Asteraceae MUH-1428	Utaa kateera	Mar. to May	W	H	A	Whole plant /tea, paste, extract	Oral and topical	Stomach problems, nerve tonic and aphrodisiac agent.	31	0.56	34	0.62
53.	*Eclipta prostrata* (L.) L. Asteraceae MUH-1405	Phol buti	May to Jul.	W	H	A	Leaf, whole plant/ juice, infusion	Oral and topical	Bacterial and fungal diseases, skin rashes, hair fall and oxidative stress.	23	0.42	35	0.64
54.	*Eruca sativa* L. Brassicaceae MUH-1274	Jaamaan	April to June	W	H	A	Leaf, seeds/ juice, infusion	Oral and topical	Body fatigue, rashes, lice killer, mosquito repellant, laxative and used as fodder for cattle and EVMs.	37	0.67	54	0.98
55.	*Euphorbia helioscopia* L. Euphorbiaceae MUH-1559	Dodal	Jan. to Apr.	W	H	A	Leaf, whole plant, seed/ extract	Oral and topical	Wormicidal, skin rashes and purgative purpose.	23	0.42	44	0.80
56.	*Euphorbia heterophylla* L. Euphorbiaceae MUH-1560	Dodal	Jan. to Oct.	W	H	A	Whole plant/ decoction	Oral and topical	Microbial disease/ infections, skin diseases and respiratory diseases.	18	0.33	42	0.76
57.	*Euphorbia hirta* L. Euphorbiaceae MUH-1561	Lailee Dodal	Jun. to Dec.	W	H	A	Seeds, leaf/ extract	Topical and oral	Diarrhea, bacterial infections, diabetics, inflammatory problems.	13	0.24	33	0.60
58.	*Euphorbia indica* Lam. Euphorbiaceae MUH-1563	Dodalee	Jun. to Sep.	W	H	A	Whole plant/decoction	Topical and oral	Snake bite, scorpion bite and immune disorders.	24	0.44	41	0.75
59.	*Euphorbia prolifera* Buch.-Ham. Euphorbiaceae MUH-1562	Dodal	Jun. to Sep.	W	H	A	Whole plant/ extract	Topical and oral	Skin diseases, anemia, kidney diseases and microbial infections.	35	0.64	42	0.76
60.	*Euphorbia prostrata* Ait. Euphorbiaceae MUH-1564	Hazaar dani	Jun. to Aug.	W	H	A	Leaf, whole plant/infusion, decoction	Oral and topical	Diuretic, cough, chest infections and vomiting.	33	0.60	32	0.58
61.	*Ficus auriculata* Lour. Moraceae MUH-1598	Pakwaree	Aug. to Nov.	W	T	P	Stem, fruit, leaf/ tea, decoction, powder	Oral, topical and gargle	Toothache, constipation, chest infections, oral infection and gastrointestinal.	44	0.80	49	0.89
62.	*Ficus benghalensis* L. Moraceae MUH-1595	Bohr	May to Jun.	W	T	P	Stem, leaf, fruit, latex/ decoction, tea	Oral, topical and gargle	Spermatogenesis, skin diseases, diabetes and toothache.	41	0.75	47	0.85
63.	*Ficus palmata* Forssk. Moraceae MUH-1597	Pakwar	May to Oct.	W	T	P	Leaf, fruit, wood/ decoction, tea	Oral, topical and gargle	Stomach disorders i.e. ulcers, and sexual disorders, diabetes, tonic, laxative and toothache.	31	0.56	43	0.78
64.	*Ficus religiosa* L. Moraceae MUH-1596	Peepal	Mar. to Apr.	W	T	P	Seed, fruit, root/ powder, tea	Oral, topical and gargle	Asthma, dysentery, diabetes, wounds healing, epilepsy, diarrhea, fever, gastritis, inflammation, infectious and sexual disorders.	33	0.60	41	0.75
65.	*Ficus semicordata* Buch.-Ham. ex Smith Moraceae MUH-1599	Pakwaree	Mar. to May	W	T	P	Fruit, bark, wood/ tea, decoction	Oral, topical and gargle	Toothache, gums bleeding, Asthma, digestive problems, skin diseases, inflammation and diabetes.	37	0.67	51	0.93
66.	*Ficus variegata* Blume Moraceae MUH-1596	Kancheer	May to Jun.	W	T	P	Leaf, fruit, bark / decoction	Oral, topical and gargle	Skin diseases, diabetes, tonic, respiratory and chest disorders, fungal allergy and toothache.	36	0.65	48	0.87
67.	*Ficus racemosa* L. Moraceae MUH-1593	Tomentosa	May to Jul.	W	T	P	Leaf, bark, fruit/tea, infusion	Oral, topical and gargle	Stomachache, diarrhea, respiratory infections, piles, diabetes, liver disorder and urinary diseases.	35	0.64	46	0.84
68.	*Flacourtia indica* (Burm. f.) Merill. Flacourtiaceae MUH-1290	Kako	Mar. to Apr.	W	T	P	Fruit, leaf /powder, tea, infusion	Oral and topical	Liver disorderes, malaria cure, snakebite and arthritis.	25	0.45	35	0.64
69.	*Fumaria indica* (Hausskn.) Pugs. Fumariaceae MUH-1270	Papra	Feb. to Jun.	W	H	A	Leaf and stem/ decoction	ORAL AND TOPICAL	BLOOD PURIFIER, DIAPHORETIC AND ANTIPYRETIC.	23	0.42	43	0.78
70.	*Gloriosa superba* L. Colchicaceae MUH-1614	Kalihari	Nov. to Apr.	W	H	A	Root, leaf/ tea, paste	Oral and Topical	Colic pains, stomachache, constipation, tumors and haemorrhoids.	23	0.42	42	0.76
71.	*Grewia optiva* J.R. Drumm. ex Burret. Tiliaceae MUH-1304	Dhaman	Apr. to Sep.	W	T	P	Stem, leaf, fruit/ tea, extract, infusion, paste	Oral and Topical	Aphrodisiac, wound healing, prolapse of placenta and as EVMs.	32	0.58	48	0.87
72.	*Ipomoea carnea* Jacq. Convolvulaceae MUH-1474	Jangli baikar	Jul. to Nov.	W	S	P	Leaf, bark/ decoction, paste	Oral and Topical	Cancer, rheumatic, purgative, wound healing and hypertension.	28	0.51	37	0.67
73.	*Ipomoea eriocarpa* R.Br. Convolvulaceae MUH-1476	Bhanwar boti	Jul. to Oct.	W	S	P	Leaf, bark, flower/ powder, tea	Oral, and Topical	Cancer and other tumors issues; eczema problems and skin diseases.	16	0.29	38	0.69
74.	*Ipomoea cairica* (L.) Sweet Convolvulaceae MUH-1479	Neeli bail	Aug. to Nov.	W	S	P	Leaf, bark/ decoction, infusion	Oral, and Topical	Fever, encephalitis, viral infections and skin problems.	18	0.33	36	0.65
75.	*Juglans regia* L. Juglandaceae MUH-1600	Akhrot	Feb. to Apr.	W	T	P	Fruit, leaf, bark/ infusion, decoction	Oral and Topical	Body tonic, constipation, teeth cleanser, chronic cough, asthma, flu, bacterial infections and dyspepsia.	45	0.82	51	0.93
76.	*Justicia adhatoda* L. Acanthaceae MUH-1505	Baikar	Aug. to Oct.	W	S	P	Leaf, bark, fruit / decoction, extract	Oral and Topical	Wound healing, septic problems, abortifacient, arthritis, chest pain, wound healing, diabetes, cancer and as EVMs.	48	42.00	55	1.00
77.	*Kickxia ramosissima* (Wall.) Janchen Scrophulariaceae MUH-1495	Khunjer buti	Mar. to Apr.	W	H	A	Leaf, bark/ decoction, tea	Oral, and Topical	Diabetes, wound healing, sores, skin irriatations, irritation, diarrhoea and cuts cure.	42	0.76	48	0.87
78.	*Kyllinga brevifolia* Rottb. Cyperaceae MUH-1669	Sedge	Aug. to Sep.	W	H	A	Leaf, bark/ infusion, extract	Oral and Topical	Inflammations, viral infections, diabetics, flu and chest infections.	41	0.75	43	0.78
79.	*Launea coromandelica* (Houtt.) Merr. Anacardiaceae MUH-1418	Kalmaan	Mar. to Jul.	W	T	P	Leaf, bark, wood/ decoction. tea	Oral, and Topical	Feet inflammations, sprains, body swellings, ulcers, elephantiasis and used as EVMs.	25	0.45	42	0.76
80.	*Launea procumbens* Roxb. Asteraceae MUH-1414	Khara Dodal	Mar. to Apr.	W	H	A	Leaf, whole plant/poultice, decoction	Oral, and Topical	Wound healing, gonorrhea, cardial pains, inflammation, cancer and broken bones.	24	0.44	33	0.60
81.	*Lindenbergia macrostachya* (Benth.) Benth. Scrophulariaceae MUH-1496	Lindlee	Mar. to Apr.	W	H	A	Leaf, stem, root/ decoction	Oral and Topical	Fever, cough, other bacterial and fungal diseases.	45	0.82	45	0.82
82.	*Loranthus longiflorus* Desr. Loranthaceae MUH-1551	Purakh	Dec. to Mar.	W	PS	P	Leaf, flower/ decoction	Oral and Topical	Diabetes, sexual infertility, cancer, skin diseases, boils, setting dislocated bones and extracting pus.	48	0.87	52	0.95
83.	*Loranthus pulverulentus* Wall. Loranthaceae MUH-1555	Phurak	Dec. to Apr.	W	PS	P	Leaf, flower/ powder, tea	Oral and Topical	Diabetes, cancer, Parkinson’s disease, coronary heart disease, skin diseases and boils.	46	0.84	50	0.91
84.	*Mallotus philipiensis* (Lamk.) Muell. Arg. Euphorbiaceae MUH-1567	Kameela	Mar. to May	W	S	P	Inflorescence, leaf/ tea, extract	Oral and Topical	Urinary issues, vulnerary, diuretic, skin disorders, heating, purgative, anthelmintic and rodents killer.	44	0.80	42	0.76
85.	*Malva parviflora* L. Malvaceae MUH-1297	Sonchal	Dec. to Mar.	W	H	A	Whole plant/poultice, decoction	Oral and Topical	Skin diseases, cough, inflammatory problems, ulcers, microbial diseases and cure of dandruff.	32	0.58	45	0.82
86.	*Malva sylvestris* L. Malvaceae MUH-1298	Sonchal	Dec. to Mar.	W	H	A	Leaf, whole plant/ decoction, tea	Oral and Topical	Stomachache, stomatitis, wormicide, glossitis, wounds healing, oral thrush and abscesses.	33	0.60	41	0.75
87.	*Malvastrum coromandelianum* (L.) Garcke Malvaceae MUH-1299	Damhni	Mar. to Dec.	W	H	A	Leaf, whole plant /decoction, extract	Oral and Topical	Aphrodisiac, chest disorders. antinociceptive, inflammation issues, analgesic and bacterial diseases.	22	0.40	35	0.64
88.	*Maytenus royleana* (Wall. ex M.A. Lawson.) Cufd. Celastraceae MUH-1324	Patakee	Feb. to Mar.	W	S	P	Fruit, seeds, leaf/ decoction, extract	Oral and Topical	Microbial infection, analgesic, gastric ulcers, inflammation problems and allergy.	43	0.78	48	0.87
89.	*Medicago polymorpha* L. Leguminosae; subfamily: Papilionaceae MUH-1347	Sareeri	Mar. to May	W	H	A	Leaf, whole plant /tea, decoction	Oral and Topical	Fever in goats/ cattle, laxative, constipation, soar throat and used as EVMs.	34	0.62	42	0.76
90.	*Medicago laciniata* var. *laciniata* L. Leguminosae; subfamily: Papilionaceae MUH-1349	Sareera	Apr. to Jul.	W	H	A	Leaf, whole plant / decoction, extract	Oral and Topical	Constipation, fever, microbial infirmities and milk yield enhancer.	42	0.76	47	0.85
91.	*Melia azedarach* (L.) Pers. Meliaceae MUH-1322	Darek	Mar. to Apr.	W	T	P	Seed, leaf bark/ decoction, poultice, tea	Oral and Topical	Asthma, blood purifier, diabetes, germicide, diuretic and used as EVMs.	45	0.82	51	0.93
92.	*Melilotus alba* L. Leguminosae; subfamily Papilionaceae MUH-1352	Methee	Mar. to Sep.	W	H	A	Leaf, whole plant/ decoction, tea	Oral and Topical	Fever, carminative, emollient, indigestion, flatulence and used as EVMs.	42	0.76	50	0.91
93.	*Melilotus indica* (L.) All. Leguminosae; subfamily Papilionaceae MUH-1350	Ran-methee	Mar. to Jul.	W	H	A	Leaf, whole plant / decoction	Oral and Topical	Diarrhea, emollient, fever, skin rash, tumors, wound healing, gastrointestinal and used as EVMs.	37	0.67	42	0.76
94.	*Mentha arvensis* L. Lamiaceae MUH-1527	Safed podina	May to Oct.	W	H	A	Leaf, whole plant/ decoction, powder, tea	Oral and Topical	Indigestion, carminative, dyspepsia, diarrhea and dysentery, stomachache, allergy and used as EVMs.	52	0.95	58	1.05
95.	*Mentha royleana* Benth. Lamiaceae MUH-1526	Jangli podia	May to Oct.	W	H	A	Leaf, whole plant/ decoction, tea	Oral and Topical	Diabetics, anticholestrol, diuretic, headache and used as EVMs.	51	0.93	61	1.11
96.	*Mentha spicata* L. Lamiaceae MUH-1525	Podina	Jul. to Aug.	W	H	A	Leaf, stem, root/ decoction, tea	Oral and Topical	Indigestion, dyspepsia, cholestrol, diuretic and headache, stomach problems and used as EVMs.	50	0.91	62	1.13
97.	*Moringa oleifera* Lam. Moringaceae MUH-1581	Sohanjna	Apr. to Jun.	W	T	P	Leaf, fruit, seed, bark/ powder, decoction	Oral and Topical	Tooth pains, stomach ulcers, asthma, diabetes, fatty liver, inflammatory problems, infertility, oxidative stress and cardiovascular issues.	49	0.89	76	1.38
98.	*Morus alba* (L.) Roxb. Moraceae MUH-1591	Safed toot	Apr. to Sep.	W	T	P	Fruit/ juice, infusion, tea	Oral and Topical	Sore throat, cough, fever, toothache and used as EVMs.	44	0.80	52	0.95
99.	*Morus macruora* Miq. Moraceae MUH-1588	Shahtoot	Mar. to Aug.	W	T	P	Leaf, fruit, wood/ juice, decoction	Oral and Topical	Sore throat, inflammatory disorders, urinary problems, cough, fever and used as EVMs.	43	0.78	58	1.05
100.	*Morus serrata* Roxb. Moraceae MUH-1589	Kancheer toot	Mar. to May	W	T	P	Leaf, fruit, wood/juice, decoction	Oral and Topical	Flu, fever and sore throat problems, disorders and urinary problems.	46	0.84	52	0.95
101.	*Morus nigra* L. Moraceae MUH-1590	Kala toot	Mar. to Jul.	W	T	P	Fruit, leaf, wood/ juiced, decoction	Oral and Topical	Anemia, cough, flu, sore throat, disorders, urinary problems and used as EVM.	41	0.75	51	0.93
102.	*Nerium oleander* L. Apocynaceae MUH-1446	Gandeera	Apr. to Sep.	W	S	P	Leaves, latex, bark/ decoction, extract	Oral and Topical	Stomach pain, skin diseases, toothache, ear and eye problems and repellant of insects.	34	0.62	41	0.75
103.	*Nicotiana plumbaginifolia* Viv. Solanaceae MUH-1491	Jangli Tomakoo	May to Jul.	W	H	A	Leaf, seed, flower/ decoction, tea	Oral and Topical	Haemorrhoids, wound healing, snake and scorpions stings’ pains.	24	0.44	42	0.76
104.	*Olea ferruginea* Wall. ex Aitch. Oleaceae MUH-1443	Kahoo	Apr. to May	W	T	P	Leaf, wood, bark/decoction	Oral and Topical	Flu, cough, jaundice and liver problems, gonorrhea, blood purifier. The branches are used as miswak (tooth brush) to cure bleeding gums and used as EVMs.	28	0.51	43	0.78
105.	*Otostegia limbata* (Bth.) Bioss. Lamiaceae MUH-1518	Chitee buti	Apr. to Aug.	W	S	P	Leaf, bark/ decoction, tea	Oral and Topical	Eye diseases and infections, ulcers, depressant, inflammation infirmities and bacterial diseases.	36	0.65	40	0.73
106.	*Oxalis corniculata* L. Oxalidaceae MUH-1318	Kati meti	Mar. to Dec.	W	H	A	Leaf, whole plant/ decoction, teac	Oral and Topical	Snake bites, diarrhea, stomach problems, urinary infections, enteritis, injuries, sprains and muscular swellings.	43	0.78	46	0.84
107.	*Papaver hybridum* L. Papaveraceae MUH-1267	Kashkash	Mar. to Jun.	W	H	A	Seeds/ powder, decoction	Oral and Topical	Weak eyes sight, pain killers and narcotic effects used as tonic for body vigour.	44	0.80	48	0.87
108.	*Papaver somnifera* L. Papaveraceae MUH-1268	Poost	Mar. to Jun.	W	H	A	Seeds, latex/ decoction, tea	Oral and Topical	Vigor tonic and sedative, dysentery, cough, brain memory enhancer and expectorant.	43	0.78	49	0.89
109.	*Persicaria barbata* var. barbata (L.) Hara Polygonaceae MUH-1549	Jor booti, Biskatali	Apr. to Sep.	W	H	A	Leaf, root, seed/ decoction	Oral and Topical	Bacterial infections, oxidative, oestrogenicity, fertility issues, colic pain, inflammations, urinary disorders, stomachache, and scabies.	45	0.82	42	0.76
110.	*Phalaris minor* L. Poaceae MUH-1652	Phumna gass	Aug. to Oct.	W	H	A	Leaf, whole plant/decoction	Oral and Topical	Admixture with cake of *Brassica compesstriss* and used as EVMs to cure of infirmities.	22	0.40	33	0.60
111.	*Phoenix sylvestris* (L.) Roxb. Arecaceae MUH-1621	Kajoor	Apr. to Sep.	W	T	P	Seed, fruit, leaf, root/ poultice, decoction	Oral and Topical	Flu, vomiting, urinary issues, bleeding nose, vertigo, sweetener and relief of unconsciousness.	34	0.62	41	0.75
112.	*Phyllanthus emblica* L. Phyllanthaceae MUH-1569	Aamla	Mar. to Jun.	W	T	P	Fruit, leaf, seed/ decoction, pickle, powder	Oral and Topical	Stomach diseases, diabetes, and kidney disorders, asthma, jaundice and used as EVMs.	48	0.87	49	0.89
113.	*Pinus roxburghii* Sarg. Pinaceae MUH-1255	Chir	Mar. to Jun.	W	T	P	Seed, Resin, leaf and bark/ decoction, tea	Oral and Topical	Pimples, tumor, and control bleeding from wounds, stomach pain, repellents of insects and mosquito.	45	0.82	53	0.96
114.	*Plantago major* L. Plantaginaceae MUH-1533	Jangli Isamgol	Aug. to Sep.	W	H	A	Leaf, seeds/ extract, tea	Oral and Topical	Pimples, wounds and sore pains, constipatuon and hypolipidemic.	44	0.80	44	0.80
115.	*Populus nigra* L. Salicaceae MUH-1604	Peepal	Apr. to May	W	H	A	Fruit, bark/ extract, tea	Oral and Topical	Cough, fever, cold, diuretic and used as EVMs.	43	0.78	46	0.84
116.	*Portulaca oleracea* L. Portulacaceae MUH-1392	Kulfa	Jun. to Sep.	W	H	A	Stem, root, leaf/decoction, tea	Oral and Topical	Constipation, febrifuge, vermifuge, bacterial infections, ulcer, inflammatory infirmities and wound-healing.	33	0.60	44	0.80
117.	*Punica granatum* L. Punicaceae MUH-1382	Darooona	Apr. to Jul.	W	S	P	Leaf, fruit, bark/ decoction, tea	Oral and Topical	Tumors, fever, cooling and tonic of the body, cough, sore throats, skin disorders anthelmintic, stomach pains and cadiotonic with hyperlepidimic effects.	44	0.80	51	0.93
118.	*Ranunculus muricatus* L. Ranunculaceae MUH-1256	Buti	Mar. to May.	W	H	A	Whole plant/ decoction	Oral and Topical	Cough, asthma, snake bite, tumor, heart related diseases, snake and scorpion bites.	42	0.76	47	0.85
119.	*Rhynchosia minima* (L.) DC. Leguminosae; subfamily Papilionaceae MUH-1339	Ran ghavara	Sep. to Oct.	W	H	A	Leaf, root, fruit/ tea, infusion	Oral and Topical	Flatulaence, indigestion, fever, whooping cough and abortificient.	45	0.82	54	0.98
120.	*Rhynchosia pseudo-cajan* Camb. Leguminosae; subfamily Papilionaceae MUH-1340	Ran bhot	May to Jun.	W	H	A	Leaf, root, fruit/ decoction, tea	Oral and Topical	Flu, fever, cough, purgative and chest infections.	46	0.84	48	0.87
121.	*Ricinus communis* L. Euphorbiaceae MUH-1568	Harnoli	Mar. to Oct.	W	H	A	Leaf, root, fruit/ decoction, tea	Oral and Topical	Skin and joints pains, diabetic drug, microbial ulcer, purgative and wormicidal.	41	0.75	47	0.85
122.	*Rubus fruticosus* Hk. Rosaceae MUH-1377	Akhray	Apr. to Oct.	W	H	A	Leaf, fruit / decoction, tea	Oral and Topical	Carminative, body tonic or vigour, sore throat, mouth bad smell and gum pains with inflammation.	43	0.78	51	0.93
123.	*Rumex dentatus* L. Polygonaceae MUH-1377	Jangli palak	Apr. to Oct.	W	H	A	Leaf, whole plant / infusion	Oral and Topical	Urinary issues, astringent. The leaf juice is applied for control of irritation of *Urtica dioica*.	38	0.69	45	0.82
124.	*Saccharum bengalensis* Retz. Poaceae MUH-1628	Sarkanda	Jul. to Sep.	W	H	A	Leaf, stem/decoction, tea	Oral and Topical	Flatulence in cattle, ear pain and used as EVMs for cattle and rodents.	22	0.40	36	0.65
125.	*Salvia plebeia* R.Br. Lamiaceae MUH-1530	Somandri Sokh	Mar. to Jun.	W	H	A	Leaf, root/decoction, infusion	Oral and Topical	Insecticidal, burnt wound’s pain reliever, piles, dysentery and used as EVMs.	34	0.62	37	0.67
126.	*Schoenoplectus litoralis* (Schrad.) Palla subsp. *thermalis* (Trabut) S.Hooper Cyperaceae MUH-1666	Dapla	Jun. to Sep.	W	H	A	Leaf, root/ powder, infusion	Oral and Topical	Carminative, bite pains, stomach worms and digestive tonic.	35	0.64	45	0.82
127.	*Schoenoplectus lacustris* (L.) Palla, subsp. *Lacustris* Cyperaceae MUH-1667	Kouna	Jun. to Sep.	W	H	A	Leaf, root, flower/ infusion	Oral and Topical	Diuretic, astringent and cure of tumors & boils.	34	0.62	44	0.80
128.	*Sida cordifolia* L. Malvaceae MUH-1301	Sidu booti	Apr. to Aug.	W	H	A	Leaf, fruit, seeds /decoction	Oral and Topical	Febrifuge, diuretic and demulcent agent, laxative and stomach pains.	22	0.40	35	0.64
129.	*Sida cordata* (Burm.f.) Borss. var. *cordata*. Malvaceae MUH-1300	Kalli buti	All year	W	H	A	Leaf, fruit / extract, poultice	Oral and Topical	Wound, cold, flu, sore mouth cough, cuts, headache, nasal congestion and diarrhea.	25	0.45	42	0.76
130.	*Sisymbrium irio* L. Brassicaceae MUH-1272	Khob Kalan	Mar. to May	W	H	A	Seeds, leaf/ decoction	Oral and Topical	Expectorant, constipation, soar throat, pharynx problems of low voice, viral flus and cure of measles.	45	0.82	34	0.62
131.	*Solanum nigrum* L. Solanaceae MUH-1484	Kach Mach	All the year	W	H	A	Leaf, fruit, root/ decoction, tea	Oral and Topical	Abortifacient, dropsy and hepatitis, kidney problems skin diseases, hepatitis, dysentery, stomachache and tumor cure.	47	0.85	37	0.67
132.	*Solanum surratense* Burm. f. Solanaceae MUH-1485	Mokari	Sep. to Mar.	W	H	A	Leaf, fruit, root/decoction, tea	Oral and Topical	Expectorant, diuretic, cure of gonorrhea, microbial infections, anti-protective, asthma, wound healing, flu, cough and fever.	35	0.64	47	0.85
133.	*Sonchus asper* L. Asteraceae MUH-1412	Kohri	Feb. to Apr.	W	H	A	Whole plant/ decoction, tea	Oral and Topical	Bacterial infections, oxidative stress and diabetes	24	0.44	35	0.64
134.	*Stellaria media* (L.) Vill. Caryophyllaceae MUH-1286	Chachunmba	Jan. to Apr.	W	H	A	Leaf, whole plant/decoction, poultice	Oral and Topical	Carminative, diuretic, laxative, expectorant, astringent and vulnerary.	42	0.76	48	0.87
135.	*Syzygium cumini* (L.) Skeels Myrtaceae MUH-1374	Jaman	Apr. to May	W	T	P	Fruit, leaf, wood/ paste, decoction, infusion	Oral and Topical	Diabetes, bronchitis, hyperglycemia, astringent helminthic, sore throat, asthma, dysentery, concomitant thirst and ulcers.	47	0.85	49	0.89
136.	*Taraxacum officinale* Weber. Asteraceae MUH-1406	Handd	Feb. to Apr.	W	H	A	Leaf, whole plant, flower/ decoction, tea	Oral and Topical	Diuretic, jaundice, heart problems, bandage with eggs as paste on broken bones, viral flu infections and wormicidal.	42	0.76	51	0.93
137.	*Terminalia belerica* (Gaertn) Roxb. Combretaceae MUH-1578	Baihra	Apr. to Jun.	W	T	P	Leaf, seed, flower, stem/ decoction, tea	Oral and Topical	Stomach and colic pains, fever, asthma and skin, haemorrhoids and diarrhea. The plant is used as source ethnoveterinary medicines (EVMs).	48	0.87	58	1.05
138.	*Toona ciliata* M.Roem Meliaceae MUH-1323	Tun	Mar. to Apr.	W	T	P	Leaf, wood, bark/ decoction, tea	Oral and Topical	Dysentery, blood diseases and stomach flatulence issues.	34	0.62	47	0.85
139.	*Trianthema portulacastrum* L. Aizoaceae MUH-1491	It-sit	Jun. to Sep.	W	H	A	Leaf, root/ decoction, paste	Oral and Topical	Stomach problems, night blindness, inflammation, constipation, laxative tonic and analgesic.	26	0.47	44	0.80
140.	*Tribulus terrestris* L Zygophyllaceae MUH-1313	Phakray	Mar. to Jul.	W	H	P	Seeds, leaf/ decoction, powder	Oral and Topical	Body tonic, impotence and vigour, urinary, cystitis problems and aphrodisiac.	41	0.75	49	0.89
141.	*Urtica dioica* L. Urticaceae MUH-1574	Bichu boti	May to Sep.	W	H	A	Leaf, root/ infusion, extract	Oral and Topical	Hay fever, jaundice, hepatitis, blood pressure, diabetes, menstrual problems and leucorrhea.	33	0.60	44	0.80
142.	*Vaccaria hispanica* (Mill.) Rauschert Caryophyllaceae MUH-1288	Masna	Feb. to Mar.	W	H	A	Whole plant/ decoction	Oral and Topical	Skin, chest tumors, menstrual disorders, enhancement of lactation in mothers and itching on the body parts.	25	0.45	36	0.65
143.	*Vallaris solanacea* (Roth) O. Kuntze Apocynaceae MUH-1288	Dhudi	Feb. to Mar.	W	H	A	Leaf, stem, root/ decoction, infusion	Oral and Topical	Skin infections, soar throat, wounds and cuts on body pains.	33	0.60	45	0.82
144.	*Viola canescens* Wall.ex Roxb. Violaceae MUH-1281	Banafsha	Mar. to Aug.	W	H	A	Flower, root/ powder, tea, extract	Oral and Topical	Flu, cold, fever, cough, soar throat, antipyretic, laxative in folklore tonics, malaria and tumors.	45	0.82	59	1.07
145.	*Withania coolgulans* L. Solanaceae MUH-1488	Paneer	Feb. to Apr.	W	H	A	Leaf, fruit / decoction, extract	Oral and Topical	Insomnia, disability and fatigue, impotence and nervous exhaustion.	54	0.98	64	1.16
146.	*Withania somnifera* (L.) Dunal. Solanaceae MUH-1487	Aksan	Feb. to Apr.	W	H	A	Fruit, leaf, root/ decoction, tea	Oral and Topical	Boils, pimples and blisters, knees pains, dyspepsia, kidney problems, rheumatism, tumors, sex potential enhancer, bacterial and mycotic infirmities.	52	0.95	68	1.24
147.	*Zanthoxylum armatum* DC. Rutaceae MUH-1319	Timbar	Mar. to Apr.	W	S	P	Seed, stem, leaf, wood /paste, decoction, infusion	Oral and Topical	Eye sights enhancer, carminative and digestives, stomachic fevers and toothache. The plant is used as source ethnoveterinary medicines (EVMs).	51	0.93	69	1.25
148.	*Ziziphus mauritiana* Lam. var. Spontanea Rhamnaceae MUH-1329	Jandi	Mar. to Sep.	W	T	P	Fruit, leaf/decoction, tea, infusion	Oral, and Topical	Obesity reducer, boils & pimples, dyspepsia, stomachache, fever, cough and used as EVMs.	47	0.85	55	1.00
149.	*Ziziphus nummularia* (Burm.f.) Wight & Arn. Rhamnaceae MUH-1328	Kokan bair	Mar. to Sep.	W	T	P	Fruit, leaf/decoction, tea	Oral and Topical	Obesity, blood purifier, diarrhea, anemia, snake biting, wound healing. The plant is used as source ethnoveterinary medicines (EVMs).	46	0.84	58	1.05
150.	*Ziziphus jujuba* Mill. Rhamnaceae MUH-1330	Unaab	Jun. to Jul.	W	T	P	Fruit, leaf/ tea, poultice, extract	Oral and Topical	Diabetes, obesity, antimicrobial, wound healing, flu, cough and used as ethnoveterinary medicines (EVMs).	39	0.71	38	0.69

The article "Ethnomedicinal and folklore inventory of wild plants used by rural communities of valley Samahni, District Bhimber Azad Jammu and Kashmir, Pakistan" was retracted in 2023. Reasons: errors in the data; errors in the methods; errors in the images; duplicated data.

### Plant part(s) used, preparation methods and mode of administration

In the study, 150 plants have been reported to be used in TEMs and many parts of the plants are used in the preparation of ethnomedicines but leaves are more prevalently used because leaf is the active area of plant machinery in which photosynthesis takes place and produces all phytoconstituents. Almost all parts of the plants are used in different TEMs, but leaves have the highest (36.49%) in usage value, followed by fruit (12.07%), whole plants (10.63%) and gum with least (4.60%) as shown in Fig 4. The similar findings have been reported in previous works conducted in in Italy and Islands which reported that the leaves were commonly used in herbal medicines [101, 102].

**Fig 4:** Percentage of plant parts used in preparation of TEMs in Samahni area of AJK.

It has been found that excessive collection of leaf along with other parts like roots and bark from plants have caused severe threats for many medicinal plants in the study area. It is also found plants’ leaves have more efficacy than other parts because leaf has more quantity of chemical constituents; furthermore potential of herbal medicine depends on use-mode, method of preparation and utilization technique [103]. There is need to start awareness campaigns to train local people about mechanism of plants’ parts collection so that medicinal plants may not be severely damaged and thrilled towards endangered and extinction zones. TEMs reported here have been prepared by using different recipes and methods such as extract, infusion, tea, decoction, powder, poultice and paste etc (Fig 5). The most common form of utilization of ethnomedicines was decoction with 29.28%, followed by tea (23.05%), extract (12.17%) and least usage form was pickle (0.66%), because pickle cannot be prepared from all parts or fruits of plants. These findings are coincident with previous works stating that decoction was the most prevalent use-form in TEMs promulgated in different areas of Pakistan [104–106] and world [107–112]. Sometime, plants are used as single recipe and sometime used as admixture in combination of different plants parts and later one is considered as the most efficient because synergistic (compound) ethnomedicines have high potential to cure infirmities [113]. Sometimes, salts or sugar are mixed with TEMs to produce better taste and aroma. Similar citations have been reported in past research works describing that decoction is prevalent mode of use [114, 115] which might be due to reason that it is easy to prepare and oral take in body [116, 117]. It is also found that decoction has more efficacy than other use-forms because it has more concentration of phytochemicals than tea or soup and same type of reports had been provided in the past publications [118, 119].

The article "Ethnomedicinal and folklore inventory of wild plants used by rural communities of valley Samahni, District Bhimber Azad Jammu and Kashmir, Pakistan" was retracted in 2023. Reasons: errors in the data; errors in the methods; errors in the images; duplicated data.

**Fig 5:** Mode of ethnomedicines used in study area, Samahni, AJK.

Although TEMs have been used in various forms but are oral administration ranked first (46.66%), followed by topical use/paste (45.92%) and gargle (10.45%) as shown in Fig 6. These findings were coincident with past works where it was stated that oral mode is preferred as it was easy to take in and also this provided instant relief from the disease [88, 120, 121]. It is reported here that use of TEMs in form of bathing and massage is also congruent with past works conducted in Gujranwala area of Pakistan. The study revealed that leaf of *Zizyphus mauritiana* and fruit of *Colocynthus lanatus* is powdered, mixed with oil and used as massage on the infirmities /pain area of body [8, 117].

**Fig 6:** Mode of administration of ethnomedicines by people of Samahni area of AJK.

### Informant consensus factor (ICF)

The informant consensus factor (ICF) was used as quantitative tool in this study to determine which infirmities were prevalent in the study area and what type of TEMs were used to cure these diseases. ICF was calculated by classifying the diseases into ten groups on the basis of the use-reports (Table 3). Among all diseases diabetics and blood pressure was ranked first with ICF value of 0.94, followed by Rabies and other sting pains (ICF: 0.93) and arthritis and joint disorders with ICF value of 0.91 (Fig 7).

**Fig 7:** Diseases prevalence with respect of use reports as per informants data of study area.

These findings confirm that ‘diabetes and blood pressure’ were the most prevalently occurring diseases in the area that might be due to excessive use of fats/butter (ghee) and change of life towards sedentary and luxurious mode. The second common type of diseases were ‘rabies and other sting pains’ followed by ‘arthritis and joint disorders’ which might be due to large occurrence of wild dogs, jackals and snakes in forest or dense plants areas of mountains of Samahni, AJK. The arthritis and knee pains were also common in the area that might be due to carrying of heavy carriage or luggage by inhabitants in form of woods and grasses to cope their daily life necessities. These findings were congruent with previous works [122–127]. The overall ICF values of the diseases occurring in the area were similar with studies conducted in different areas of Pakistan [90, 128] and Azad Kashmir [129, 130].

The article "Ethnomedicinal and folklore inventory of wild plants used by rural communities of valley Samahni, District Bhimber Azad Jammu and Kashmir, Pakistan" was retracted in 2023. Reasons: errors in the data; errors in the methods; errors in the images; duplicated data.

### Relative frequency of citation (RFC) and use value index (UVI)

The relative frequency of citation (RFC) and use value index (UVI) tools were applied to explore and determine the medicinal potential of plants and their potential for future pharmacological research and drug development. RFC confirmed the medicinal importance and acceptability of MPs with frequency of citations in the study area to cure various diseases. The RFC of medicinal plants species of the study area ranged from 0.22 to 0.95 (Table 3). The highest RFC (0.95) was found for *Acacia modesta* Wall., followed by *Boerhavia procumbens* Banks ex. Roxb. (RFC = 0.87), *Berberis lycium* Royle. (RFC = 0.85), *Ficus auriculata* Lour. (RFC = 0.83), *Carissa opaca* Stapf ex. Haines. (RFC = 0.80) and *Calotropis procera* (Aiton) Dryand (RFC = 0.75). The use value index (UVI) was calculated to find the relative importance of plants and their families in the local communities. The highest UVI was found for *Moringa oleifera* Lam. (1.38 value), followed by *Zanthoxylum armatum* DC. (1.25), *Withania somnifera* (L.) Dunal. (1.24), *Withania coolgulans* L. (1.16), *Mentha spicata* L. (1.13), *Terminalia belerica* (Gaertn) Roxb. (1.03) and *Justicia adhatoda* L. (1.00), respectively.

*Rhynchosia minima* (L.) DC. (0.97 value) and *Loranthus longiflorus* Desr. (0.95 value) as shown in Table 3. The higher values of index of UV determines that plants species are extensively used by the indigenous people for curing of different ailments. This is indication of popularity of the local medicinal flora in local culture. The plants which have low value of UVI confirms that these are less available in the area or those have less ethnomedicinal uses in the area. These findings are comparatively similar with previous studies of different areas of Pakistan. It has been reported that *Withania somnifera* (L.) Dunal. as used for cure of rheumatism, tumors, *Ziziphus nummularia* was used for treatment of stings and skin allergies. It is stated that *Solanum surratense* has many TEMs uses in local culture of the study area. Similar findings had been found in other studies of previous publications that the plant was known very medicinal in many traditional ethnomedicines [120–130]. Another plant *Withania somnifera* had also very effective TEM uses in local communities of the study area to cure sex and pregnancy problems [41]. *Solanum nigrum* is very important medicinal species being used in local folklore phytonyms and these findings are in congruent with past works [40, 41]. High values of RFC and UVI for these and other medicinal plants proved that these plants were prevalently known as medicinal plants of the area.

The article "Ethnomedicinal and folklore inventory of wild plants used by rural communities of valley Samahni, District Bhimber Azad Jammu and Kashmir, Pakistan" was retracted in 2023. Reasons: errors in the data; errors in the methods; errors in the images; duplicated data.

### Fidelity level (FL), relative popularity level (RPL), rank order of priority (ROP)

The fidelity level (FL), relative popularity level (RPL) and rank order of priority (ROP) indices were determined for 33 most predominant plants having highly medicinal values occurring in the study area (Table 4). FL of the plants ranged between 70% to100%; in which *Phyllanthus emblica* L. had 100% FL which was used to cure hypertension, hyperlipidemia; *Melia azedarach* (L.) Pers. had FL of 100%, *Solanum surattense* Burm.f. had 100% FL and these were used to cure gonorrhea, fever and least values of FL (70%) were explored for *Nerium oleander* L. which was used to cure stomachache, skin rashes in local therapeutics. High values of FL indicates the prevalence of specific disease(s) in the local area and common use of the medicinal plants for curing these diseases [41, 129]. The findings were coincide with previous results of research works which stated that medicinal plants had been playing significant role in cure of many diseases in rural areas of Pakistan [122, 123].

**Table 4:** List of indigenous plants depicting highest therapeutic uses with FL, RPL, ROP from Samahni area of District Bhimber, Azad Jammu and Kashmir.

	Plant Species	Therapeutic Uses	N	NA	FL	RPL	ROP
1.	*Phyllanthus emblica* L.	Antihypertension, Antihyperlepidemic	80.0	80.0	100.0	1.0	100
2.	*Morus macruora* Miq.	Cure Cough, Chest infection	75.0	73.0	97.3	1.0	97
3.	*Justicia adhatoda* L.	Diabetic, bacterial infection	78.0	69.0	88.5	1.0	89
4.	*Melia azedarach* (L.) Pers.	Diabetic, blood problems	80.0	80.0	100.0	1.0	96
5.	*Solanum surattense* Burm.f.	Gonorrhea, Fever	65.0	65.0	100.0	0.9	92
6.	*Solanum nigrum* L.	Hepatitis, spleen disorders	60.0	55.0	91.7	0.9	81
7.	*Ficus racemosa* L.	Piles, Constipation	55.0	52.0	94.5	0.9	80
8.	*Ziziphus nummularia* (Burm.f.) Wight & Arn.	Skin disorder, anemia	45.0	42.0	93.3	0.8	76
9.	*Ficus palmata* Forssk.	Stomachache, constipation,	44.0	41.0	93.2	0.8	73
10.	*Flacourtia indica* (Burm. f.) Merr.	Jaundice, Liver disorder	43.0	38.0	88.4	0.8	66
11.	*Albizia lebbeck* (L.) Benth.	Kidney diseases	38.0	34.0	89.5	0.7	59
12.	*Azadirachta indica* A. Juss.	Syphilis, wormicide	37.0	36.0	97.3	0.6	62
13.	*Calotropis procera* (Aiton) Dryand.	Snake and scorpion bite	31.0	26.0	83.9	0.6	52
14.	*Carissa opaca* Stapf ex Haines.	jaundice and hepatitis	28.0	22.0	78.6	0.6	46
15.	*Datura innoxia* Mill.	Flatulence, epilepsy	22.0	19.0	86.4	0.5	47
16.	*Nerium oleander* L.	Stomachache, skin rashes	20.0	14.0	70.0	0.5	32
17.	*Eruca sativa* L.	Boils and pus blisters	15.0	11.0	73.3	0.3	24
18.	*Flacourtia indica* (Burm. f.) Merill.	Antihypertension, colic, eye sight enhancer	73.0	73.0	100.0	1.0	100.0
19.	*Mentha arvensis* L.	Vigour enhancer, stomachache	77.0	73.0	94.8	1.0	94.8
20.	*Ajuga bracteosa* Wall ex Benth	Asthma, fever, hypertension	71.0	65.0	91.5	1.0	91.5
21.	*Bombax ceiba* L.	Anti-inflammation, menstrual disorders	77.0	75.0	97.4	1.0	93.5
22.	*Withania somnifera* (L.) Dunal.	Liver disorders, kidney pain, blood purifier	80.0	80.0	100.0	0.9	92.0
23.	*Ziziphus jujuba* Mill.	Diabetes, Skin disorder	65.0	64.0	98.5	0.9	86.6
24	*Ficus variegata* Blume	Eyes diseases, diabetes	55.0	51.0	92.7	0.9	78.8
25	*Olea ferruginea* Wall. ex Aitch.	Gums and teeth diseases, diabetes	71.0	71.0	100.0	0.8	81.0
26	Toona ciliata *M*.*Roem*	Haemorrhoids, diarrhoea and flatulence	66.0	65.0	98.5	0.8	76.8
27.	*Bauhinia variegata* L.	Hemorrhoids and jaundice	62.0	55.0	88.7	0.8	66.5
28.	*Punica granatum* L.	Skin and hair problems	55.0	52.0	94.5	0.7	62.4
29.	*Citrullus colocynthis* (L.) Shard	Syphilis and amenorrhea	45.0	41.0	91.1	0.6	56.5
30.	*Allium jacquemontii* Kunth	Snake and scorpion poison lecuoderma	52.0	45.0	86.5	0.6	55.4
31.	*Amaranthus viridis* L.	Constipation and inflammation	26.0	24.0	92.3	0.5	49.8
32.	*Persicaria barbata* var. barbata (L.) Hara	Skin diseases, scabies	20.0	18.0	90.0	0.5	40.5
33.	*Mentha spicata* L	Toothache and headache	19.0	16.0	84.2	0.3	28

The informants provided ethnomedicinal data of 150 plants and on basis of relative priority level (RPL) 33 important diseases’ groups and highly medicinal plants of the area were prioritized in matrix form (Table 4). There is strong correlation between number of informants describing the particular plant species and number of usages as ethnomedicine (Fig 8) and there is also significant relationship between the number of informants citing the particular plant to cure a particular disease as described in Fig 9. It is known that number of uses increases when number of informants rises because of correlation coefficient factor r = 0.10. For example, if one plant species is cited by more 25 or more informants as ethnomedicine; the number of its relative popularity level (RPL) is ranked as raised and RPL is determined as percentage of (I_u_ /25) assigned score one (1) if cited or mentioned by the half or more number (12) of total informants (25) for any disease treatment and it is ranked as popular (P). If any plant is cited by less than 12 informants then RPL value will be ranked as unpopular (UP) (Amjad *et al*., 2017). The marginalized values between P and UP of the plant is point where if informants number is increased then number of medicinal uses per plant species does not rise. These two tools of ethnobotany are commonly used for determination of commonly use-ness in the local area for cure of diseases.

The article "Ethnomedicinal and folklore inventory of wild plants used by rural communities of valley Samahni, District Bhimber Azad Jammu and Kashmir, Pakistan" was retracted in 2023. Reasons: errors in the data; errors in the methods; errors in the images; duplicated data.

**Fig 8:** Depicting correlationship between number of informants and number of TEMs use.

**Fig 9:** Depicting correlationship between numbers of uses of plant and particular disease.

The protocol of “popular (P) and unpopular (UP)” demarcates plants into main two categories with reference of their cure potential for a specific disease. Out of one hundred and fifty medicinal plants; 33 plants species were selected for FL, RPL and ROP indices and highest RPL value (1.00) was found for *Phyllanthus emblica* L., *Morus macruora* Miq., *Justicia adhatoda* L., *Melia azedarach* (L.) Pers., and *Ajuga bracteosa* Wall ex Benth. each (Fig 10) which proved that these plants were the most popular source of TEMs in the study area. The high RPL values of these plant species may be referred to their significant medicinal potential and similarly the awareness and reliability of the local people on these medicinal plants. These findings are in consistent with past studies about the medicinal plants of different areas of the Pakistan [124] and world [125, 126, 129, 130].

**Fig 10:** Diagram depicting relationship between number of respondents who told TEMs use of particular plant and its use number. Dark black area is depicting its RPL value.

The third quantitative index Rank order priority (ROP) was used for validation and confirmation of medicinal qualities of the plants reported by indigenous communities of Samahni area. This index is correlated with FL & RPL and it may be assigned the name of correction factor, primarily used when FL values are different from RPL. The RPL and FL values along with ROP are presented in Table 4. It was explored that ROP values ranged between 24–100 and out of thirty three species of plants 26 species had more than 50 values of ROP. The highest ROP (100) was found for *Phyllanthus emblica* L. and *Flacourtia indica* (Burm. f.) Merill., followed by *Morus macruora* Miq. (with 97.0 ROP value) which were reported to be used to cure hypertension and hyperlipidemia and cough, chest infection, respectively. The least ROP value (24) was found for *Eruca sativa* L. The higher ROP values than 50 means that these plants were predominantly used in local therapeutics and TEMs in the study area. The plant *Justicia adhatoda* L. had ROP of 89 and was used to treat diabetes and bacterial infections, while *Solanum surattense* Burm.f. with ROP of 92 was used to cure gonorrhea and fever. These findings were inlined with previous research works conducted on ethnomedicinal studies in different regions of Pakistan [87] and world [124, 129]. The low ROP of some reported plants in this study indicate that either these plants might be not easily available in the area or people use these plants less due to certain unknown reasons. This demands to do further ethnopharmacological and conservation work in the area to protect and conserve these medicinal plants which will also assist in documentation and preservation of bioculture and traditional ethnobotanical knowledge of the indigenous communities.

The article "Ethnomedicinal and folklore inventory of wild plants used by rural communities of valley Samahni, District Bhimber Azad Jammu and Kashmir, Pakistan" was retracted in 2023. Reasons: errors in the data; errors in the methods; errors in the images; duplicated data.

### Relative importance of plants and relative pharmaceutical significance of the most commonly used indigenous plants

In this parameter, drug development prospective and potential of the medicinal plants (MPs) is calculated by using formula of relative importance of plants (RIP) which is based on its relative pharmacological (reh. Ph.) properties of a species and body systems (BS) cured. Moreover, the multiple use of these MPs as agricultural products (agro-uses) with trade potential was also determined to prove their multiple-use, popularity and financial impact on life of local communities of the study areas (Table 5). The studies revealed that ethnopharmacological potential was described by using RIP which ranged between: 20.4 to 90.8. The highest RIP (90.80) was found for *Azadirachta indica* A. Juss. with good number of agro-uses and its seeds and bark were sold in local markets and used in herbal therapeutics by indigenous practioners. Followed by *Justicia adhatoda* L. with RIP (90.4) and *Juglans regia* L. having RIP: 88.3 while least RIP value (20.4) was found for *Cynodon dactylon* (L.) Pers. It was determined that MPs having less RIP values means that these plants have less medicinal or ethnopharmacological uses in TEMs in the study area. The other plants like: *Phyllanthus emblica* L. (RIP:80), *Terminalia arjuna* L. (RIP: 83.3), *Zanthoxylum armatum* DC. (RIP:79.6), *Moringa oleifera* Lam. (RIP:87.8) and *Morus macruora* Miq. (RIP: 79.2) depicted that these have high popularity in indigenous medicinal therapeutics and they can be declared are potential plants species for further ethnopharmacological pharmaceutical analysis to discover drug for infirmities treatment at larger scale. These findings are congruent with previous works [27, 28, 58, 62].

**Table 5:** Relative importance of plants and relative pharmaceutical significance of the most commonly used indigenous plants by the local people of different areas of Samahni, AJK, Pakistan and agro use and export status.

S No	Botanical Names	No. Ph.	Rel. Ph.	No. BS	Rel. BS.	RIP	Agro Use	Trade
01.	*Acacia modesta* Wall.	12	0.3	6	0.4	35.0	Y	Y
02.	*Acacia nilotica* (L.) Delile	9	0.2	7	0.5	34.6	Y	Y
03.	*Achyranthus aspera* L.	24	0.6	9	0.6	60.0	N	Y
04.	*Aerva sanguinolenta* (L.) Blume	25	0.6	11	0.7	67.9	N	Y
05.	*Ajuga bracteosa* Wall ex Benth.	28	0.7	13	0.9	78.3	N	Y
06.	*Albizia lebbeck* (L.) Benth.	7	0.2	10	0.7	42.1	Y	N
07.	*Allium jacquemontii* Kunth	9	0.2	8	0.5	37.9	N	N
08.	*Aloe vera* (L.) Burm. f.	23	0.6	13	0.9	72.1	N	Y
09.	*Alternanthera pungens* L.	22	0.6	11	0.7	64.2	N	N
10.	*Amaranthus viridis* L.	15	0.4	9	0.6	48.8	N	N
11.	*Artemisia scoparia* Waldst. & Kit.	16	0.4	9	0.6	50.0	N	N
12.	*Artemisia vulgaris* L.	18	0.5	8	0.5	49.2	N	N
13.	*Azadirachta indica* A. Juss.	38	1.0	13	0.9	90.8	Y	Y
14.	*Bauhinia variegata* L.	33	0.8	12	0.8	*81*.*3*	Y	Y
15.	*Berberis lycium* Royle.	23	0.6	11	0.7	65.4	N	Y
16.	*Boerhavia procumbens* Banks ex Roxb.	31	0.8	12	0.8	78.8	N	Y
17.	*Boerhavia diffusa* L.	36	0.9	10	0.7	78.3	N	Y
18.	*Bombax ceiba* L.	12	0.3	6	0.4	35.0	Y	N
19.	*Bromus japonicus* L.	9	0.2	7	0.5	34.6	N	N
20.	*Butea monosperma* (Lam.) Taub.	15	0.4	5	0.3	35.4	Y	N
21.	*Calotropis procera* (Aiton) Dryand.	24	0.6	8	0.5	56.7	N	N
22.	*Capparis decidua* (Forssk.) Edgew.	26	0.7	6	0.4	52.5	N	N
23.	*Capparis sepiaria* L.	24	0.6	9	0.6	60.0	N	N
24.	*Carissa opaca* Stapf ex Haines.	29	0.7	11	0.7	72.9	N	N
25.	*Caryopteris odorata* (D. Don) B. Rob.	12	0.3	8	0.5	41.7	N	N
26.	*Celtis eriocarpa* Decne.	14	0.4	5	0.3	34.2	N	Y
27.	*Cuscuta reflexa* Roxb.	18	0.5	4	0.3	35.8	N	N
28.	*Casearia tomentosa* Roxb.	16	0.4	7	0.5	43.3	N	N
29.	*Cassia fistula* L.	13	0.3	7	0.5	39.6	Y	N
30.	*Cenchrus biflorus* Roxb.	11	0.3	5	0.3	30.4	N	N
31.	*Ceropegia bulbosa* L.	18	0.5	8	0.5	49.2	N	N
32.	*Chenopodium album* L.	26	0.7	6	0.4	52.5	N	N
33.	*Cichorium intybus* L.	15	0.4	5	0.3	35.4	N	N
34.	*Cirsium arvensis* (L.) Scop.	22	0.6	6	0.4	47.5	N	N
35.	*Citrullus colocynthis* (L.) Shard	27	0.7	8	0.5	60.4	N	Y
36.	*Clematis grata* Wall.	23	0.6	9	0.6	58.8	N	Y
37.	*Clematis graveolens* Lindl.	21	0.5	11	0.7	62.9	N	N
38.	*Clematis connata* DC.	20	0.5	10	0.7	58.3	N	N
39.	*Colebrookea oppositifolia* Smith.	19	0.5	9	0.6	53.8	N	N
40.	*Commelina benghalensis* L.	22	0.6	6	0.4	47.5	N	Y
41.	*Convolvulus arvensis* L.	11	0.3	5	0.3	30.4	N	N
42.	*Corchorus olitorius* L.	14	0.4	4	0.3	30.8	N	N
43.	*Cordia gharaf* (Forssk.) Ehren. ex Asch	15	0.4	7	0.5	42.1	N	N
44.	*Cordia obliqa* L.	27	0.7	9	0.6	63.8	Y	Y
45.	*Cymbopogan citratus* (John) Schutt	22	0.6	4	0.3	40.8	N	N
46.	*Cynodon dactylon* (L.) Pers.	11	0.3	2	0.1	20.4	N	N
47.	*Datura innoxia* Mill	28	0.7	8	0.5	61.7	N	N
48.	*Datura stramonium* L.	29	0.7	9	0.6	66.3	N	N
49.	*Digera muricata* (L.) Mart.	22	0.6	5	0.3	44.2	N	N
50.	*Eruca sativa*	27	0.7	6	0.4	53.8	N	N
51.	*Euphorbia helioscopia* L.	22	0.6	7	0.5	50.8	N	N
52.	*Euphorbia heterophylla* L.	11	0.3	4	0.3	27.1	N	N
53.	*Euphorbia hirta* L.	8	0.2	6	0.4	30.0	N	N
54.	*Euphorbia indica* Lam.	8	0.2	7	0.5	33.3	*N*	*N*
55.	*Euphorbia prolifera* Buch.-Ham.	9	0.2	6	0.4	31.3	N	N
56.	*Euphorbia prostrata* Ait.	11	0.3	4	0.3	27.1	N	N
57.	*Ficus auriculata* Lour.	25	0.6	8	0.5	57.9	Y	Y
58.	*Ficus benghalensis* L.	28	0.7	9	0.6	65.0	Y	Y
59.	*Ficus palmata* Forssk.	20	0.5	7	0.5	48.3	Y	Y
60.	*Ficus religiosa* L.	17	0.4	8	0.5	47.9	Y	Y
61.	*Ficus semicordata* Buch.-Ham. ex Sm.	28	0.7	9	0.6	65.0	Y	Y
62.	*Ficus variegata* Blume	26	0.7	6	0.4	52.5	Y	Y
63.	*Ficus racemosa* L.	25	0.6	8	0.5	57.9	Y	Y
64.	*Flacourtia indica* (Burm. f.) Merill.	22	0.6	11	0.7	64.2	Y	N
65.	*Fumaria indica* (Hausskn.) Pugs.	25	0.6	11	0.7	67.9	N	N
66.	*Gloriosa superba* L.	23	0.6	10	0.7	62.1	N	N
67.	*Galium aparine* L.	16	0.4	12	0.8	63.4	N	N
68.	*Grewia optiva* J.R. Drumm. ex Burret	29	0.7	14	0.9	79.2	Y	N
69.	*Ipomoea carnea* Jacq.	22	0.6	11	0.7	64.2	N	N
70.	*Ipomoea eriocarpa* R.Br.	25	0.6	8	0.5	57.9	N	N
71.	*Ipomoea cairica* (L.) Sweet	23	0.6	9	0.6	58.8	N	N
72.	*Juglans regia* L.	36	0.9	13	0.9	88.3	Y	Y
73.	*Justicia adhatoda* L.	35	0.9	14	0.9	90.4	Y	N
74.	*Kickxia ramosissima* (Wall.) Janchen	12	0.3	8	0.5	41.7	N	N
75.	*Kyllinga brevifolia* Rottb.	11	0.3	4	0.3	27.1	N	N
76.	*Launea procumbens* Roxb.	22	0.6	12	0.8	67.5	N	N
77.	*Lindenbergia macrostachya* (Bth.) Bth.	16	0.4	6	0.4	40.0	N	N
78.	*Loranthus longiflorus* Desr.	15	0.4	5	0.3	35.4	N	N
79.	*Loranthus pulverulentus* Wall.	22	0.6	7	0.5	50.8	N	N
80.	*Mallotus philipiensis* (Lamk.) Mll. Arg.	25	0.6	4	0.3	44.6	Y	N
81.	*Malva parviflora* L.	22	0.6	7	0.5	50.8	N	N
82.	*Malva sylvestris* L.	12	0.3	5	0.3	31.7	N	N
83.	*Malvastrum coromandelianum* (L.) Gk	22	0.6	8	0.5	54.2	N	N
84.	*Maytenus Royleana* (W.ex.Laws.) Cudf.	23	0.6	7	0.5	52.1	Y	N
85.	*Medicago polymorpha* L.	24	0.6	5	0.3	46.7	N	N
86.	*Medicago laciniata var*. *laciniata* L.	12	0.3	4	0.3	28.3	N	N
87.	*Melia azedarach* (L.) Pers.	29	0.7	11	0.7	72.9	Y	Y
88.	*Melilotus alba* L.	23	0.6	10	0.7	62.1	N	N
89.	*Melilotus indica* (L.) All.	22	0.6	6	0.4	47.5	N	N
90.	*Mentha arvensis* L.	31	0.8	8	0.5	65.4	N	N
91.	*Mentha royleana* Benth.	32	0.8	9	0.6	70.0	N	N
92.	*Mentha spicata* L.	34	0.9	9	0.6	72.5	N	Y
93.	*Moringa oleifera* Lam.	31	0.8	12	0.8	78.8	Y	Y
94.	*Morus macruora* Miq.	34	0.9	11	0.7	79.2	Y	Y
95.	*Morus alba* (L.) Roxb.	29	0.7	12	0.8	76.3	Y	Y
96.	*Morus serrata* Roxb.	25	0.6	10	0.7	64.6	Y	Y
97.	*Morus nigra* L.	26	0.7	12	0.8	72.5	Y	N
98.	*Nerium oleander* L.	16	0.4	10	0.7	53.3	Y	N
99.	*Nicotiana plumbaginifolia* Viv.	12	0.3	8	0.5	41.7	N	N
100.	*Olea ferruginea* Wall. ex Aitch.	28	0.7	11	0.7	71.7	Y	N
101.	*Otostegia limbata* (Bth.) Bioss.	22	0.6	8	0.5	54.2	N	N
102.	*Oxalis corniculata* L.	24	0.6	9	0.6	60.0	N	N
103.	*Papaver hybridum* L.	25	0.6	7	0.5	54.6	N	N
104.	*Papaver somnifera* L.	23	0.6	9	0.6	58.8	N	Y
105.	*Persicaria barbata* (L.) Hara	26	0.7	11	0.7	69.2	N	N
106.	*Phalaris minor* L.	21	0.5	4	0.3	39.6	N	N
107.	*Phoenix sylvestris* (L.) Roxb.	24	0.6	8	0.5	56.7	N	N
108.	*Phyllanthus emblica* L.	32	0.8	12	0.8	80.0	Y	Y
109.	*Pinus roxburghii* Sargent	33	0.8	9	0.6	71.3	Y	Y
110.	*Plantago major* L.	28	0.7	5	0.3	51.7	N	N
111.	*Populus nigra* L.	20	0.5	11	0.7	61.7	N	Y
112.	*Portulaca oleracea* L.	16	0.4	6	0.4	40.0	N	N
113.	*Punica granatum* L.	18	0.5	9	0.6	52.5	N	N
114.	*Ranunculus muricatus* L.	13	0.3	4	0.3	29.6	N	N
115.	*Rhynchosia minima* (L.) DC.	22	0.6	5	0.3	44.2	N	N
116.	*Rhynchosia pseudo-cajan* Camb.	24	0.6	9	0.6	60.0	N	N
117.	*Ricinus communis* L.	22	0.6	5	0.3	44.2	N	N
118.	*Rubus fruticosus* Hk.	11	0.3	6	0.4	33.8	N	N
119.	*Rumex dentatus* L.	12	0.3	7	0.5	38.3	N	N
120.	*Saccharum bengalensis* Retz.	9	0.2	8	0.5	37.9	N	N
121.	*Salvia plebeia* R.Br.	5	0.1	5	0.3	22.9	N	N
122.	*Saussurea heteromalla* (Don)Hand. Mz	14	0.4	9	0.6	47.5	N	N
123.	*Schoenoplectus lacustris* (L.) Palla	19	0.5	5	0.3	40.4	N	N
124.	*Schoenoplectus litoralis* (Schrad.) Palla subsp. *thermalis* (Trabut) S.Hooper	22	0.6	6	0.4	47.5	N	N
125.	*Sida cordifolia* L.	12	0.3	3	0.2	25.0	N	N
126.	*Sida cordata* (Burm.f.) Borss.	14	0.4	5	0.3	34.2	N	N
127.	*Sisymbrium irio* L.	19	0.5	9	0.6	53.8	N	Y
128.	*Solanum nigrum* L.	30	0.8	8	0.5	64.2	N	Y
129.	*Solanum surattense* Burm. f.	31	0.8	5	0.3	55.4	N	Y
130.	*Sonchus asper* L.	22	0.6	7	0.5	50.8	N	N
131.	*Stellaria media* (L.) Vill.	12	0.3	7	0.5	38.3	N	N
132.	*Syzygium cumini* (L.) Skeels	27	0.7	8	0.5	60.4	N	Y
133.	*Taraxacum officinale* Weber.	29	0.7	12	0.8	76.3	N	N
134.	*Terminalia arjuna* L.	34	0.9	11	0.7	82.9	Y	Y
135.	*Terminalia belerica* (Gaertn) Roxb.	32	0.8	13	0.9	83.3	Y	Y
136.	*Toona ciliate* M. Roem	12	0.3	4	0.3	28.3	Y	N
137.	*Trianthema portulacastrum* L.	21	0.5	5	0.3	42.9	N	N
138.	*Tribulus terrestris* L.	25	0.6	7	0.5	54.6	N	N
139.	*Urtica dioica* L.	21	0.5	5	0.3	42.9	N	N
140.	*Vaccaria hispanica* (Mill.) Rauschert	12	0.3	3	0.2	25.0	N	N
141.	*Vallaris solanacea (Roth) O*. *Kuntze*	11	0.3	4	0.3	27.1	N	N
142.	*Verbascum thapsus* L.	15	0.4	2	0.1	25.4	N	N
143.	*Verbena officinalis* L.	16	0.4	4	0.3	33.3	N	Y
144.	*Viola canescens* Wall.ex Roxb.	34	0.9	12	0.8	82.5	N	Y
145.	*Withania coolgulans* L.	34	0.9	9	0.6	72.5	N	Y
146.	*Withania somnifera* (L.) Dunal.	32	0.8	11	0.7	76.7	N	Y
147.	*Zanthoxylum armatum* DC.	29	0.7	13	0.9	79.6	Y	Y
148.	*Ziziphus mauritiana* Lam. var. Spontanea	22	0.6	12	0.8	67.5	Y	Y
149.	*Ziziphus nummularia* (Burm.f.) W.A.	29	0.7	11	0.7	72.9	Y	N
150.	*Ziziphus jujuba* Mill.	26	0.7	9	0.6	62.5	Y	N

The article "Ethnomedicinal and folklore inventory of wild plants used by rural communities of valley Samahni, District Bhimber Azad Jammu and Kashmir, Pakistan" was retracted in 2023. Reasons: errors in the data; errors in the methods; errors in the images; duplicated data.

### Innovation and future prospective of research

The current research is the first quantitative study comprising of 150 plant species used in traditional ethnomedicines (TEMs) in rural mountainous area of Samahni, District Bhimber of Azad Jammu and Kashmir, Pakistan. The study is very innovative as it is first quantitative ethnomedicinal research work conducted on prevalently used plants in TEMs in the study area. These ethnomedicinal findings are compared with previous research works conducted in District Bhimber of Azad Kashmir [3, 6, 19, 31, 32–34] other parts of AJK [114–117, 119, 120] and different areas of Pakistan [121–130]. As medicinal plants reported here are first time properly documented and authenticated using quantitative statistical tools and many of these wild plants are first time reported here in this study as medicinal species. The key importance of this research is that it has different recipes with mode of use determined by RPL, ROP and ICF which contains famous folklore phytotherapeutics *viz*: *Clematis connata* DC. (boils and tumors), *Cordia gharaf* (Forssk.) Ehren ex. Asch. (fever, cough, diuretic, demulcent, stomachache), *Echinochola crus-galli* L. (spleen disorders, skin allergies), *Ficus palmata* Forssk. (stomachache, diabetes, toothache), *Flacourtia indica* (Burm.f.) Merill. (liver disorderes, antimalarial), *Allium jacquemontii* Kunth. (snake bite, sting of scorpion) and *Aloe vera* (L.) Burm. f. (piles, anal irritation, diabetics, baldness, wound healing, skin diseases). In this study, the plants species with high RPL and FL values might be recommended for further phytochemical and ethnopharmacological research to discover novel drugs and produce allopathic drugs at industrial level by using pharmaceutical research protocols to cope with emerging resistant pathogenic microbes for safe and better health of human beings. Future conservation work for rare medicinal plants species of the area is urgent need of time.

## Conclusion and recommendations

The current study confirms that TEMs obtained from plants are major source of medication used by rural and mountainous communities of the Samahni area of AJK, Pakistan. The local people hitherto are dependent on “green or botanic drugs” obtained from wild flora of the area. Although allopathic medicines are available in nearby District headquarters but still majority of the people prefer to use TEMs to cure different infirmities because indigenous people consider that botanic drugs are easy to collect and prepare, cheap, nontoxic and have better synergistic impact for treatment of chronic and acute diseases. This research work will provide the foundation linkage among rural dwellers, local herbalists and scientific researchers because it may lead towards discovering of neo-medicines through dedicated procedures and conservation of biocultural heritage by documentation. Following recommendations are suggested with future perspectives: (i) to document and preserve traditional ethnomedicines of the area as booklet form and analyze their dose optimization using latest protocols, (ii) to do further ethnopharmacological research on plants with high RPL, RFC and ROP to discover novel drugs (iii) to conserve rare and threatened medicinal plants of the area by using dedicated approaches involving concerned departments and indigenous people of the area, (iv) to provide practice measures for sustainable utilization of wild natural resources of the study and (v) to optimize and recommend herbal medicines to cure neo-emerging Covid-19 causing massive loss of lives around the globe. This and similar type of ethnomedicinal studies will make a pathway for discovering of novel drugs for mitigation and eradication of such fatal pandemic of Covid-19 through public message and track-path for future researchers.

The article "Ethnomedicinal and folklore inventory of wild plants used by rural communities of valley Samahni, District Bhimber Azad Jammu and Kashmir, Pakistan" was retracted in 2023. Reasons: errors in the data; errors in the methods; errors in the images; duplicated data.

## Supporting information

S1 Questionnaire (DOCX)
